The article "A multiple attribute group decision making model based on 2-tuple linguistic pythagorean fuzzy dombi aggregation operators for optimal selection of potential global suppliers" was published in 2024. Journal: Heliyon.

# A multiple attribute group decision making model based on 2-tuple linguistic pythagorean fuzzy dombi aggregation operators for optimal selection of potential global suppliers

**DOI:** 10.1016/j.heliyon.2024.e34570

**Published:** 2024-07-20

**Authors:** Tmader Alballa, Ahmed Alamer, Khadija Nasir, Awais Yousaf, Somayah Abdualziz Alhabeeb, Hamiden Abd El-Wahed Khalifa

**Affiliations:** a Department of Mathematics, College of Sciences, Princess Nourah Bint Abdulrahman University, P.O. Box 84428, Riyadh, 11671, Saudi Arabia; b Department of Mathematics, Faculty of Science University of Tabuk, Tabuk, 71491, Saudi Arabia; c Department of Mathematics, The Islamia University of Bahawalpur, 63100, Bahawalpur, Pakistan; d Department of Mathematics, College of Science, Qassim University, Buraydah, 51452, Saudi Arabia; e Department of Operations and Management Research, Faculty of Graduate Studies for Statistical Research, Cairo University, Giza, 12613, Egypt

**Keywords:** 2-Tuple linguistic pythagorean fuzzy numbers, Dombi operations, 2TLPFDWA aggregation operators, 2TLPFDWG aggregation operators, Multiple attribute group decision making

## Abstract

Multiple-Attribute Group Decision-Making (MAGDM) is a significant area of research in decision-making, and its principles and methodologies are widely implemented. A Pythagorean Fuzzy Set (PFS) is an extension of an Intuitionistic Fuzzy Set (IFS) that is highly valuable for representing uncertain information in real-world scenarios. The 2-Tuple Linguistic Pythagorean Fuzzy Number (2TLPFN) is a specific type of Pythagorean Fuzzy Number (PFN) that can be used to represent uncertainty in real-world decision making through the use of 2-Tuple Linguistic Terms (2TLTs). This paper focuses on the examination of Multiple Attribute Group Decision Making (MAGDM) using 2TLPFNs. Dombi's t-norm and t-conorm operations were commonly referred to as Dombi operations, which might have been greater degree of applicability if offered in a new form of flexibility within the general parameter. In this research, we implement Dombi operations to construct some 2-Tuple Linguistic Pythagorean Fuzzy (2TLPF) Dombi Aggregation operators. These operators include the 2TLPF Dombi Weighted Averaging (2TLPFDWA) operator, 2TLPF Dombi Ordered Weighted Averaging (2TLPFDOWA) operator, 2TLPF Dombi Weighted Geometric (2TLPFDWG) operator, and 2TLPF Dombi Ordered Weighted Geometric (2TLPFDOWA) operator. An analysis is conducted to examine the unique characteristics of these suggested operators. Subsequently, we leveraged the proposed operators to develop a model aimed at tackling the MAGDM problems in the 2TLPF environment. Eventually, a suitable instance has been demonstrated to validate the formation of the model as well as exhibit its implementation and resilience.

The article "A multiple attribute group decision making model based on 2-tuple linguistic pythagorean fuzzy dombi aggregation operators for optimal selection of potential global suppliers" was published in 2024. Journal: Heliyon.

## 1 Introduction

The investigation of Multiple Attribute Group Decision Making (MAGDM) problems in the context of linguistic data processing systems has become a captivating subject of research, attracting growing interest in recent years. Atanassov's IFS however generalizes over the basic principles of mathematical analysis of fuzzy sets. IFS is a better and more realistic approach of giving the inherent fuzziness into the data with both the membership as well as non-membership degrees. Several IFS aggregation operators has been developed within the last few decades [1]. However, in the modern world, the recent development of the PFSs (Possibility Fuzzy Sets) has been used to solve the problem of uncertainty in Multiple Attribute Decision Making (MADM) environments. Therefore, PFS distinguishes itself as a membership degree (MD), and the non-membership degree (NMD), the former's total with the latter squared being less than or equal to 1. There are instances where PFS has effectiveness in addressing various matters that IFS is ineffective in dealing with. For example if an authority suggests that the values for MD and NMD are 0 then it simply cannot be accepted. 8 and 0. and IFS, respectively: hence while the concept of PFS will be able to manage this situation the concept of IFS will possibly not be able to. Also, it is proved that all IFS degrees are included in PFS degrees, which suggests that PFSs have better mechanisms to deal with the uncertainty.

It is imperative to note that the 2TLPFNs are a special case of the Pythagorean Fuzzy Numbers (PFNs). Among the successful models applied in the linguistic data processing, one of the most noteworthy is the 2-tuple linguistic computational model [2]. This model has demonstrated that through the use of 2- tuples, the cause of minimized losses and distortions in the processing of linguistic data is successfully achieved. The authors listed several operators like the 2TAA operator, 2TWA operator, 2TOWA operator, and E2TWA operator by Herrerra et al. [3]. Herrera et al. [b] claimed that a framework accepted and deals with the calculation of non-homogeneous information. In their work, Herrera et al. [4] proposed a paradigm for consistency support in terms of multiple-granularity preference relations. Liao et al. [5] employed linguistic data for selecting an ERP system. In an effort to develop the model of fuzzy language which made room for word sets in language that are unevenly distributed, Herrera et al. [6]. Wang [7] proposed a 2TLF assessment approach with the goal of determining the best appropriate option. Tai et al. [8] made a valuable contribution by developing a linguistic component as part of the intellectual capital assessment methodology. Fan et al. [9] adopted a Fuzzy Linguistic Method to assess the proficiency of firms in managing information. Wei developed the TOPSIS methodology for Multiple Attribute Group Decision Making (MAGDM), integrating the 2 TL data. Wei proposed the ET−WG and ET−OWG operators to aid with MAGDM procedures that utilize 2 TL data. Fan (2015) proposed a framework for uncertain linguistic decision making that incorporates many levels of granularity. In addition, Chang and Wen [10] developed a very effective and distinctive 2TOWA operator in the context of DFMEA. Also, Jiang et al. [11] proposed the use of Bonferroni Mean operations to incorporate two-tuple linguistic knowledge. Xu et al. [12] developed many methods to handle unwanted imperfect 2-tuple fuzzy language preference connections in instances when decisions are made collectively. Liu et al. [13] established DI2TL aggregation operators for the purpose of selecting decisions within various attribute groups. Dutta et al. [14] developed a framework based on linguistic 2-tuples to handle attribute heterogeneity in MADM. In addition, Dong et al. [15] created a synthetic framework that focuses on consistency to establish interval numerical scales for 2TLTs. This strategy was employed in a linguistic GDM environment, specifically focusing on a preference relation. The method devised by Wang et al. [16] revolves around the utilization of I2TL data and the application of Choquet Integral aggregation operators. Qin and Liu [17] also advocated the implementation of 2TLMMOs in MAGDM and applied this in the course of supplier selection. Furthermore, Zhang, Xu, and Wang [18] proposed the MAGDM under the CRM with the help of 2-Tuple linguistic information. Their interest was on cases whereby weight data is Inadequate. PFSs that have a degree of 4–5 has been identified as a feasible approach in AS concerning MADM issues on Ambiguity. PFS has its special memberships and non-memberships which states that it is better suited for more purposes as compared to IFSs. According to PFS, there are certain difficulties which IFS cannot address clearly; as such, PFS also proves how it is able to cope with ambiguous problems. PFNs were defined by Zhang and Xu [19] while Zhang and Xu [19] also introduced a comprehensive equation of PFS. Moreover, they put forward the implementation of a Pythagorean Fuzzy TOPSIS to respond to multiple criteria decision-making difficulties in Pythagorean Fuzzy Networks. Besides, Peng and Yang [20] have put forward the employing of the division and subtraction operations related to PFN and Pythagorean Fuzzy differentiation between the processes for superiority and inferiority rating for solving MCGDM issues with PFNs. In this study, ‘averaging’ of PFNs has been discussed as one of the aggregation functions and after conducting the experiment it was established that the averaging aggregation function gives results that match standard fuzzy numbers. Reformat et al. [21] employed PFNs to handle a collaborative recommendation system. Gou et al. [22] analyzed the attributes of CPF data. In addition, Ren et al. [23] proposed the Pythagorean fuzzy TODIM technique for multiple criteria decision making (MCDM), whereas Garg [24] applied averaging Einstein Operations to create Generalized Pythagorean Fuzzy Information Aggregation. PFS has the ability to tackle challenges that IFS is unable to manage, highlighting its effectiveness in resolving ambiguous problems. Wei et al. [25] proposed the notion of P2TLSs and P2TL data aggregation techniques. In their study, Deng et al. [26] proposed the concept of 2TLPFSs and provided some Hamy mean procedures that can be used to them. Deng et al. [27] developed a collection of Bonferroni mean operations employing 2TLPFSs. Deng et al. [28] devised the CODAS method for 2TLP fuzzy MAGDM and implemented it in the assessment of financial management performance.

The article "A multiple attribute group decision making model based on 2-tuple linguistic pythagorean fuzzy dombi aggregation operators for optimal selection of potential global suppliers" was published in 2024. Journal: Heliyon.

Seikh et al. [29] introduced some picture fuzzy aggregation operators based on Frank t-norm and t-conorm and their application to MADM process. Therefore, Seikh et al. [30] introduced the q-Rung Orthopair Fuzzy Archimedean aggregation operators. Dombi [31] created the more flexible Dombi t−norm and Dombi t−conorm by a parameter in aggregation process. Dombi t-norm and t-conorm are often considered more important or advantageous than Frank/Archimedean t-norm and t-conorm in contexts where flexibility, smooth transitions, intuitive adjustability, and broad applicability are critical. The parameterized nature of Dombi operations provides a high degree of adaptability and fine-tuning, making them suitable for a wide range of applications and better able to model complex systems with varying interaction dynamics. Archimedean t-norms and t-conorms, while valuable and covering a broad range of operations, do not offer the same level of intuitive control and smooth transition as Dombi operations. The averaging/geometric operations assist in converting the data into a single value. Dombi operators solve decision-making problems with great effectiveness and remarkable adaptability to operational circumstances. Seikh et al. [32] introduced the IF Dombi aggregation operators and their application to MADM. Further, Seikh et al. [33] introduced the Interval-valued Fermatean fuzzy Dombi aggregation operators and SWARA based PROMETHEE II method to bio-medical waste management. Mandal et al. [34] introduced the Interval-valued Spherical Fuzzy MABAC method based on Dombi aggregation operators with unknown attribute weights to select plastic waste management process. Zhang et al. [35] introduced the MADM technique using Single-valued Neutrosophic Trigonometric Dombi aggregation operators.

The article "A multiple attribute group decision making model based on 2-tuple linguistic pythagorean fuzzy dombi aggregation operators for optimal selection of potential global suppliers" was published in 2024. Journal: Heliyon.

According to the previous study, most of the existing 2TLPF aggregation strategies include using the algebraic sum and product of 2TLPFSs to carry out the aggregation process. However, none of these aggregation algorithms consider the specific connections between the variables being combined. In order to address this limitation and drawing inspiration from the Dombi average and Dombi geometric operations, we present a set of 2TLPFDW Arithmetic/Geometric Aggregation Operators in this work.

### 1.1 Motivations

The following are the key motivations for this work.

1. The 2-tuple linguistic model and the prominent characteristics of PFSs are combined in a single formulation to create the 2TLPFSs, an innovative information representation model. We may simply represent the aggregated MD and NMD values in a predefined linguistic term set (LTS) by using the 2-tuple linguistic Pythagorean fuzzy information model. Consequently, the research work being done in 2TLPF environment can be attributed to the nature of the 2TLPFSs.
2. Some of the merits of Dombi aggregation operators include the following; It can incorporate blurred and obscure pieces of information. It can be used flexibly in various decision-making environments on the basis of variation in the decision-maker's risk-taking appetite. To meet the requirements of different consumers, they combine realistic elements with some degree of positive outlook and eliminate strict adherence to recklessness. Dombi operators are the mediators between numerical and language data and gives output in common language; they work on any type of data – quantitative or qualitative. Furthermore, they are efficient means when it comes to solving a number of practical problems because of a relative flexibility of these models which enables to better coordinate and thus make more rational decisions. In the context of this study, the set of aggregation operators for 2TLPF data is novel and developed precisely for processing the information with the help of powerful Dombi operations and the flexibility of the 2TLPFSs construct. These operators provide a stable and flexible framework to agglomerate the process using the powerful aspect of Dombi operations and extending the advanced modelling features of 2TLPFSs.
3. In the real society there arises many decision making problems, which involve distinct processes and information, which is often ambiguous and uncertain, therefore decision making theory must develop fresh MAGDM. Several limitations can be envisaged with the current methodologies for MAGDM in the 2TLPF when it comes in managing group decision-making issues when the weights of the attributes are fully unknown.

The article "A multiple attribute group decision making model based on 2-tuple linguistic pythagorean fuzzy dombi aggregation operators for optimal selection of potential global suppliers" was published in 2024. Journal: Heliyon.

### 1.2 Objectives

1. Identify simple arithmetic operations for 2 TLPFSs based on Dombi geometry. This has also involved development of mathematical structures to define how distinct 2TLPFS components communicate and hence better event assessment which translates to better estimates.
2. More information on 2TLPFD aggregation operators should be collected and 2TLPFD aggregation operators should be studied. As a result, this will entail finding out how several 2TPFD operators can be combined in order to arrive at more effective 2TLPFS aggregation methods.
3. While new operators are defined, features which differentiate them from the previous ones should be emphasized. The elaborated characteristics, in connection with the proposed operators, will be substantiated by means of profound mathematical analysis and step-by-step descriptions.
4. Propose a solution method employing the 2TLPFD aggregation operators to solve MAGDM issues. This will also logically include developing a systematic way of solving and evaluating complex decision making issues using the new operators.
5. Based on the newly blended technique identify the best potential supplier in supply chain management. That will require applying the suggested approach to problem situations.
6. Present a comparison analysis to show the suggested technique's validity when compared to existing approaches. The suggested method's effectiveness will be tested against existing methods using data from real-life situations and scenarios.

### 1.3 Contributions

1. The PythagoreanFuzzySets(PFSs) represent membership degree and non-membership degree, utilizing numerical values ranging from 0 to 1. The 2TLPFSs contain the levels of membership and non-membership, which are enclosed under the 2 TL model. Addressing real-world MAGDM issues in which experts communicate their perspectives using language concepts is more beneficial.
2. The suggested operators demonstrate remarkable adaptability. Their effectiveness applies not just to 2TLPF data, but furthermore includes 2TLIF data, therefore avoiding the restrictions of already present operators.
3. This article presents an introduction and study of the 2TLPFDWA, 2TLPFDOWA, 2TLPFDWG, and 2TLPFDOWG operators including a comprehensive examination of their key features.
4. A variety of fields, such as multi-criteria decision evaluation, data extraction, systems for making decisions, and more, can benefit from the ideas covered in this discussion. This cross-disciplinary applicability makes the contributions relevant not just for scholars in the discipline of aggregation technique but also for professionals who seek efficient methods for real-world issues in diverse disciplines.
5. A computational structure for MAGDM created from 2TLPF dataset is provided in order to optimize the best choice from the restricted range of possibilities. Implementing the suggested methodologies leads to a thorough solution, thereby assessing the quality and feasibility of the given strategy.
6. Finally, an unbiased examination shows that the suggested aggregation operators are legitimate and effective. The primary aim of this project is to provide a more attractive combined operator for addressing problems with numerous attributes, together with a more efficient and systematic approach for communicating evaluation results. Moreover, the capacity to adaptively modify parameters allows for the flexibility to generate diverse choice outcomes considering the choice maker's risk viewpoint under various risk scenarios.

The article "A multiple attribute group decision making model based on 2-tuple linguistic pythagorean fuzzy dombi aggregation operators for optimal selection of potential global suppliers" was published in 2024. Journal: Heliyon.

List of abbreviations is presented in Table 1.

**Table 1:** List of abbreviations.

Abbreviations	Meanings
MADM	Multiple Attribute Decision Making
MAGDM	Multiple Attribute Group Decision Making
DMs	Decision Makers
MD	Membership Degree
NMD	Non-membership Degree
FST	Fuzzy Set Theory
2TLTs	2-Tuple Linguistic Terms
IFSs	Intuitionistic Fuzzy Sets
PFSs	Pythagorean Fuzzy Sets
2TLPFSs	2-Tuple Linguistic Pythagorean Fuzzy Sets
AOs	Aggregation Operators
2TLPFDWAA	2TLPF Dombi Weighted Averaging Aggregation
2TLPFDWA	2TLPF Dombi Weighted Averaging
2TLPFDOWA	2TLPF Dombi Ordered Weighted Averaging
2TLPFDWGA	2TLPF Dombi Weighted Geometric Aggregation
2TLPFDWG	2TLPF Dombi Weighted Geometric
2TLPFDOWG	2TLPF Dombi Ordered Weighted Geometric
SCM	Supply Chain Management

The rest of this article is organized as follows: In Sect. 2, we introduce some basic concepts of 2 TL representation model, PFSs, 2TLPFSs and Dombi operators, including definitions, properties, and working rules. In Sect. 3, we propose Dombi Operations on 2TLPFNs. In Sect. 4, we propose several operators 2TLPFDWA, 2TLPFDOWA, 2TLPFDWG, and 2TLPFDOWG with certain specific features. In Sec. 5, the proposed AOs are used to build the MAGDM model. Sec. 6 provides a numerical example of potential global supplier selection using 2TLPNs to demonstrate the technique described in this article. Section 7 contains the conclusions.

The article "A multiple attribute group decision making model based on 2-tuple linguistic pythagorean fuzzy dombi aggregation operators for optimal selection of potential global suppliers" was published in 2024. Journal: Heliyon.

## 2 Preliminaries

Based on the PFSs and 2−TupleLinguisticTerms(2TLTs), We present a brief explanation of many important ideas and theories of 2TLPFSs.

### 2.1 A linguistic terms set (LTS)

#### 2.1.1 **Definition 2.1.1** [36,37]

Let $E=\{{ɇ}_{i}|\;i=0,1,2,\ldots ,\tau \}$ be a LTS with odd cardinality, where ${ɇ}_{i}$ denotes a feasible value for a language-based variable that meets the following requirements:

1) hesetisordered:${ɇ}_{i}>{ɇ}_{j},if\;i>j$;
2) $\mathrm{Max}\;operator:\max\left({ɇ}_{i},{ɇ}_{j}\right)={ɇ}_{i},if\;{ɇ}_{i}\geq {ɇ}_{j}$;
3) $\mathrm{Min}\;operator:\min\left({ɇ}_{i},{ɇ}_{j}\right)={ɇ}_{i},if\;{ɇ}_{i}\leq {ɇ}_{j}$.

For example, E can be defined as

$$E=\left\{{ɇ}_{0}=extremely\;poor,{ɇ}_{1}=very\;poor,{ɇ}_{2}=poor,{ɇ}_{3}=slightly\;poor,{ɇ}_{4}=fair,{ɇ}_{5}=slightly\;good,{ɇ}_{6}=good,{ɇ}_{7}=very\;good,{ɇ}_{8}=extremely\;good\right\}\text{.}$$

### 2.2 A 2-tuple linguistic (2 TL) model

#### 2.2.1 Definition 2.2.1 [36]

Let $E=\{{ɇ}_{i}|\;i=0,1,2,\ldots ,\tau \}$ be a LTS. A pair $\left({ɇ}_{i},\mu \right)$ representing language terms ${ɇ}_{i}$ and a numeric value (μ) is known as symbolic translation. It represents the fuzzy membership function's translation and displays the nearest term ${ɇ}_{i}\in \left\{{ɇ}_{0},{ɇ}_{1},\ldots ,{ɇ}_{\tau }\right\}$. This is the 2 TL model. The definition of $\mu^{\prime }s$ value is defined in Eq (1):

(1) $$\mu =\left\{ \begin{array}{c} {}[-\frac{1}{2},\frac{1}{2}),if\;{ɇ}_{i}\in \left\{{ɇ}_{0},{ɇ}_{1},\ldots ,{ɇ}_{\tau -1}\right\},\\ {}[0,\frac{1}{2}),if\;{ɇ}_{i}={ɇ}_{o},\\ {}[-\frac{1}{2},0),if\;{ɇ}_{i}={ɇ}_{\tau }.\; \end{array}\right.$$

#### 2.2.2 Definition 2.2.2 [36]

Let $E=\{{ɇ}_{i}|\;i=0,1,2,\ldots ,\tau \}$ be a LTS, and ω∈[0,τ]. Then the function Δ which is utilized to transform ω into a 2-tuple is defined in Eq (2):

$$\Delta :\left[0,\tau \right]\to E\times [-\frac{1}{2},\frac{1}{2})\text{.}$$

(2) $$\Delta \left(\omega \right)=\left({ɇ}_{i},\mu \right)\;\text{with}\;\left\{ \begin{array}{c} {ɇ}_{i},i=\text{round}\left(\omega \right),\\ \mu =\omega -i,\mu \in [-\frac{1}{2},\frac{1}{2}). \end{array}\right.$$

where, round (.) denotes the usual round operation.

#### 2.2.3 Definition 2.2.3 [36]

Let $E=\{{ɇ}_{i}|\;i=0,1,2,\ldots ,\tau \}\text{,}$ be a LTS and consider $\left({ɇ}_{i},\mu \right)$ is a 2‐tuple, then there exists an inverse function $\Delta^{-1\;}$, which can transform a 2-tuple to its nearest numerical value ω∈[0,τ]. The inverse function $\Delta^{-1\;}$ is defined in Eq (3):

$$\Delta^{-1\;}:E\times [-\frac{1}{2},\frac{1}{2})\to \left[0,\tau \right]$$

(3) $$\Delta^{-1}\left({ɇ}_{i},\mu \right)=i+\mu =\omega \text{.}$$

#### 2.2.4 Definition 2.2.4 [36]

Let $\left({ɇ}_{u},\mu_{1}\right)$ and $\left({ɇ}_{v},\mu_{2}\right)$ be two 2−tuplelinguistic values. Then,

1. If $u<v,then\;\left({ɇ}_{u},\mu_{1}\right)<\left({ɇ}_{v},\mu_{2}\right)$.
2. If u<v,then.
  a) If $\mu_{1}=\mu_{2},then\;\left({ɇ}_{u},\mu_{1}\right)=\left({ɇ}_{v},\mu_{2}\right)$.
  b) If $\mu_{1}<\mu_{2},then\;\left({ɇ}_{u},\mu_{1}\right)<\left({ɇ}_{v},\mu_{2}\right)$.
  c) If $\mu_{1}>\mu_{2},then\;\left({ɇ}_{u},\mu_{1}\right)>\left({ɇ}_{v},\mu_{2}\right)$.

The article "A multiple attribute group decision making model based on 2-tuple linguistic pythagorean fuzzy dombi aggregation operators for optimal selection of potential global suppliers" was published in 2024. Journal: Heliyon.

### 2.3 A Pythagorean Fuzzy Set (PFS)

#### 2.3.1 Definition [38,39]

In the world of discourse Y, a PythagoreanfuzzysetP is an object having the form presented in Eq (4):

(4) $$P=\left\{\left(y,\left(\alpha_{P}\left(y\right),\beta_{P}\left(y\right)\right)|y\in Y\right)\right\}\text{.}$$

where.

a. ($\alpha_{P}\left(y\right)):Y\to \left[0,1\right])\text{,}$ express the membership degree function for every y in P.
b. ($\left(\beta_{P}\left(y\right)):Y\to \left[0,1\right]\right)\text{,}$ express the non-membership degree function for every y in P.

Where, the criteria are satisfied by the degree of membership and non-membership $0\leq {\left(\alpha_{P}\left(y\right)\right)}^{2}+{\left(\beta_{P}\left(y\right)\right)}^{2}\leq 1\text{,}$ for all y∈Y.

### 2.4 A 2-tuple linguistic Pythagorean Fuzzy Set (2TLPFS)

#### 2.4.1 Definition [27]

Let $E=\{{ɇ}_{i}|\;i=0,1,2,\ldots ,\tau \}$ be a set of linguistic terms with odd cardinality τ+1. If $\left(\left({ɇ}_{u}\left(y\right),£\left(y\right)\right),\left({ɇ}_{v}\left(y\right),ℵ\left(y\right)\right)\right)$ is defined for $({ɇ}_{u}\left(y\right),({ɇ}_{v}\left(y\right)\in E$ and $£\left(y\right),ℵ\left(y\right)\in [-\frac{1}{2},\frac{1}{2})$, where $\left({ɇ}_{u}\left(y\right),£\left(y\right)\right)$ and $\left({ɇ}_{v}\left(y\right),ℵ\left(y\right)\right))$ represent the MD and NMD by 2TLTs, respectively. A 2TLPFS is defined in Eq (5):

(5) $$¥=\left\{y,\left(\left({ɇ}_{u}\left(y\right),£\left(y\right)\right),\left({ɇ}_{v}\left(y\right),ℵ\left(y\right)\right)\right)\;|y\in Y\right\}\text{.}$$

where, ${0\leq \Delta }^{-1}\left({ɇ}_{u}\left(y\right),£\left(y\right)\right)\leq \tau ,{0\leq \Delta }^{-1}\left({ɇ}_{v}\left(y\right),ℵ\left(y\right)\right)\leq \tau$, satisfying the condition presented in Eq (6):

$$0\leq {\left(\Delta^{-1}\left({ɇ}_{u}\left(y\right),£\left(y\right)\right)\right)}^{2}+{\left(\Delta^{-1}\left({ɇ}_{v}\left(y\right),ℵ\left(y\right)\right)\right)}^{2}\leq \tau^{2}\text{.}$$

(6) $$0\leq {\left(\frac{\Delta^{-1}\left({ɇ}_{u}\left(y\right),£\left(y\right)\right)}{\tau }\right)}^{2}+{\left(\frac{\Delta^{-1}\left({ɇ}_{v}\left(y\right),ℵ\left(y\right)\right)}{\tau }\right)}^{2}\leq 1\text{.}$$

#### 2.4.2 Definition [27]

Let $¥=\left(\left({ɇ}_{u},£\right),\left({ɇ}_{v},ℵ\right)\right)$ be a set of 2TLPFNs. Then, the definition of the score function of ¥ is given in Eq (7):

(7) $${€}_{S}\left(¥\right)=\Delta \left(\frac{\tau }{2}\left(1+{\left(\frac{\Delta^{-1}\left({ɇ}_{u},£\right)}{\tau }\right)}^{2}-{\left(\frac{\Delta^{-1}\left({ɇ}_{v},ℵ\right)}{\tau }\right)}^{2}\right)\right),{€}_{S}\left(¥\right)\in \left[0,\tau \right]\text{.}$$

The definition of the accuracy function for ¥, which is given in Eq (8):

(8) $${€}_{H}\left(¥\right)=\Delta \left(\tau \left({\left(\frac{\Delta^{-1}\left({ɇ}_{u},£\right)}{\tau }\right)}^{2}+{\left(\frac{\Delta^{-1}\left({ɇ}_{v},ℵ\right)}{\tau }\right)}^{2}\right)\right),{€}_{H}\left(¥\right)\in \left[0,\tau \right]\text{.}$$

The article "A multiple attribute group decision making model based on 2-tuple linguistic pythagorean fuzzy dombi aggregation operators for optimal selection of potential global suppliers" was published in 2024. Journal: Heliyon.

#### 2.4.3 Definition [27]

Let ${¥}_{1}=\left(\left({ɇ}_{u_{1}},{£}_{1}\right),\left({ɇ}_{v_{1}},{ℵ}_{1}\right)\right)\text{,}$ and ${¥}_{2}=\left(\left({ɇ}_{u_{2}},{£}_{2}\right),\left({ɇ}_{v_{2}},{ℵ}_{2}\right)\right)$ be any two 2TLPFNs. Then,

1. If ${€}_{s}\left({¥}_{1}\right)<{€}_{s}\left({¥}_{2}\right),then\;{¥}_{1}<{¥}_{2}$.
2. If ${€}_{s}\left({¥}_{1}\right)>{€}_{s}\left({¥}_{2}\right),then{¥}_{1}{>¥}_{2}$.
3. If ${€}_{s}\left({¥}_{1}\right)={€}_{s}\left({¥}_{2}\right),then$.
  (a) If ${€}_{H}\left({¥}_{1}\right)>{€}_{H}\left({¥}_{2}\right),then{¥}_{1}>{¥}_{2}$.
  (b) If ${€}_{H}\left({¥}_{1}\right)<{€}_{H}\left({¥}_{2}\right),then{¥}_{1}<{¥}_{2}$.
  (c) If ${€}_{H}\left({¥}_{1}\right)={€}_{H}\left({¥}_{2}\right),then{¥}_{1}={¥}_{2}$.

#### 2.4.4 Definition [27]

Let $¥=\left(\left({ɇ}_{u},£\right),\left({ɇ}_{v},ℵ\right)\right)\text{,}$ ${¥}_{1}=\left(\left({ɇ}_{u_{1}},{£}_{1}\right),\left({ɇ}_{v_{1}},{ℵ}_{1}\right)\right)\text{,}$ and ${¥}_{2}=\left(\left({ɇ}_{u_{2}},{£}_{2}\right),\left({ɇ}_{v_{2}},{ℵ}_{2}\right)\right)$ are three 2TLPFNs, and ϕ>0, then some basic operations of the 2TLPFNs are designed as follows:

1. ${¥}_{1}⊕{¥}_{2}=\left(\begin{array}{c} \Delta \left(\tau \sqrt[{2}]{{\left(\frac{\Delta^{-1}\left({ɇ}_{u_{1}},{£}_{1}\right)}{\tau }\right)}^{2}+{\left(\frac{\Delta^{-1}\left({ɇ}_{u_{2}},{£}_{2}\right)}{\tau }\right)}^{2}-{\left(\frac{\Delta^{-1}\left({ɇ}_{u_{1}},{£}_{1}\right)}{\tau }\right)}^{2}.{\left(\frac{\Delta^{-1}\left({ɇ}_{u_{2}},{£}_{2}\right)}{\tau }\right)}^{2}}\right),\\ \Delta \left(\tau \left(\frac{\left(\Delta^{-1}\left({ɇ}_{v_{1}},{ℵ}_{1}\right)\right)}{\tau }.\frac{\left(\Delta^{-1}\left({ɇ}_{v_{2}},{ℵ}_{2}\right)\right)}{\tau }\right)\right) \end{array}\right)$.
2. ${¥}_{1}⊗{¥}_{2}=\left(\begin{array}{c} \Delta \left(\tau \left(\frac{\Delta^{-1}\left({ɇ}_{u_{1}},{£}_{1}\right)}{\tau }.\frac{\Delta^{-1}\left({ɇ}_{u_{2}},{£}_{2}\right)}{\tau }\right)\right),\\ \Delta \left(\tau \sqrt[{2}]{{\left(\frac{\Delta^{-1}\left({ɇ}_{v_{1}},{ℵ}_{1}\right)}{\tau }\right)}^{2}+{\left(\frac{\Delta^{-1}\left({ɇ}_{v_{2}},{ℵ}_{2}\right)}{\tau }\right)}^{2}-{\left(\frac{\Delta^{-1}\left({ɇ}_{v_{1}},{ℵ}_{1}\right)}{\tau }\right)}^{2}.{\left(\frac{\Delta^{-1}\left({ɇ}_{v_{2}},{ℵ}_{2}\right)}{\tau }\right)}^{2}}\right) \end{array}\right)$.
3. $\phi .¥=\left(\begin{array}{c} \Delta \left(\tau \sqrt[{2}]{\left(1-{\left(1-{\left(\frac{\Delta^{-1}\left({ɇ}_{u},£\right)}{\tau }\right)}^{2}\right)}^{\phi }\right)}\right),\\ \Delta \left(\tau {\left(\frac{\Delta^{-1}\left({ɇ}_{v},ℵ\right)}{\tau }\right)}^{\phi }\right) \end{array}\right)$.
4. ${¥}^{\phi }=\left(\begin{array}{c} \Delta \left(\tau {\left(\frac{\left({ɇ}_{u},£\right)}{\tau }\right)}^{\phi }\right),\\ \Delta \left(\tau \sqrt[{2}]{\left(1-{\left(1-{\left(\frac{\Delta^{-1}\left({ɇ}_{v},ℵ\right)}{\tau }\right)}^{2}\right)}^{\phi }\right)}\right) \end{array}\right)$.

The article "A multiple attribute group decision making model based on 2-tuple linguistic pythagorean fuzzy dombi aggregation operators for optimal selection of potential global suppliers" was published in 2024. Journal: Heliyon.

## 3 Dombi Operations on 2TLPFNs

### 3.1 Definition [31]

The definition of Dombi t−norm for two real numbers mandn is defined in Eq (9):

(9) $$T^{Dom}\left(m,n\right)=\frac{1}{1+{\left\{{\left(\frac{1-m}{m}\right)}^{d}+{\left(\frac{1-n}{n}\right)}^{d}\right\}}^{\frac{1}{d}}}\text{.}$$

Thus, the definition of Dombi t−conorm for two real numbers mandn is defined in Eq (10):

(10) $$S^{Dom}\left(m,n\right)=1-\frac{1}{1+{\left\{{\left(\frac{m}{1-m}\right)}^{d}+{\left(\frac{n}{1-n}\right)}^{d}\right\}}^{\frac{1}{d}}}\text{.}$$

where, (m,n)∈[0,1]×[0,1] and d>0.

### 3.2 Definition

Let $¥=\left(\left({ɇ}_{u},£\right),\left({ɇ}_{v},ℵ\right)\right)\text{,}$ ${¥}_{1}=\left(\left({ɇ}_{u_{1}},{£}_{1}\right),\left({ɇ}_{v_{1}},{ℵ}_{1}\right)\right)\text{,}$ and ${¥}_{2}=\left(\left({ɇ}_{u_{2}},{£}_{2}\right),\left({ɇ}_{v_{2}},{ℵ}_{2}\right)\right)$ are three 2TLPFNs, and ϕ>0, then some Dombi t−norm and Dombi t−conorm operational laws for 2TLPFNs are designed as follows;

1. ${¥}_{1}⊕{¥}_{2}=\left(\begin{array}{c} \Delta \left(\tau -\frac{\tau }{1+{\left\{{\left(\frac{\Delta^{-1}\left({ɇ}_{u_{1}},{£}_{1}\right)}{\tau -\Delta^{-1}\left({ɇ}_{u_{1}},{£}_{1}\right)}\right)}^{\gamma }+{\left(\frac{\Delta^{-1}\left({ɇ}_{u_{2}},{£}_{2}\right)}{\tau -\Delta^{-1}\left({ɇ}_{u_{2}},{£}_{2}\right)}\right)}^{\gamma }\right\}}^{\frac{1}{\gamma }}}\right),\\ \Delta \left(\frac{\tau }{1+{\left\{{\left(\frac{\tau -\Delta^{-1}\left({ɇ}_{v_{1}},{ℵ}_{1}\right)}{\Delta^{-1}\left({ɇ}_{v_{1}},{ℵ}_{1}\right)}\right)}^{\gamma }+{\left(\frac{\tau -\Delta^{-1}\left({ɇ}_{v_{2}},{ℵ}_{2}\right)}{\Delta^{-1}\left({ɇ}_{v_{2}},{ℵ}_{2}\right)}\right)}^{\gamma }\right\}}^{\frac{1}{\gamma }}}\right) \end{array}\right)$.
2 ${¥}_{1}⊗{¥}_{2}=\left(\begin{array}{c} \Delta \left(\frac{\tau }{1+{\left\{{\left(\frac{\tau -\Delta^{-1}\left({ɇ}_{u_{1}},{£}_{1}\right)}{\Delta^{-1}\left({ɇ}_{u_{1}},{£}_{1}\right)}\right)}^{\gamma }+{\left(\frac{\tau -\Delta^{-1}\left({ɇ}_{u_{2}},{£}_{2}\right)}{\Delta^{-1}\left({ɇ}_{u_{2}},{£}_{2}\right)}\right)}^{\gamma }\right\}}^{\frac{1}{\gamma }}}\right),\\ \Delta \left(\tau -\frac{\tau }{1+{\left\{{\left(\frac{\Delta^{-1}\left({ɇ}_{v_{1}},{ℵ}_{1}\right)}{\tau -\Delta^{-1}\left({ɇ}_{v_{1}},{ℵ}_{1}\right)}\right)}^{\gamma }+{\left(\frac{\Delta^{-1}\left({ɇ}_{v_{2}},{ℵ}_{2}\right)}{\tau -\Delta^{-1}\left({ɇ}_{v_{2}},{ℵ}_{2}\right)}\right)}^{\gamma }\right\}}^{\frac{1}{\gamma }}}\right) \end{array}\right)$.
3 $\phi .¥=\left(\begin{array}{c} \Delta \left(\tau -\frac{\tau }{1+{\left\{\phi {\left(\frac{\Delta^{-1}\left({ɇ}_{u},£\right)}{\tau -\Delta^{-1}\left({ɇ}_{u},£\right)}\right)}^{\gamma }\right\}}^{\frac{1}{\gamma }}}\right),\\ \Delta \left(\frac{\tau }{1+{\left\{{\phi \left(\frac{\tau -\Delta^{-1}\left({ɇ}_{v},ℵ\right)}{\Delta^{-1}\left({ɇ}_{v},ℵ\right)}\right)}^{\gamma }\right\}}^{\frac{1}{\gamma }}}\right) \end{array}\right)$.
4 ${¥}^{\phi }=\left(\begin{array}{c} \Delta \left(\frac{\tau }{1+{\left\{\phi {\left(\frac{\tau -\Delta^{-1}\left({ɇ}_{u},£\right)}{\Delta^{-1}\left({ɇ}_{u},£\right)}\right)}^{\gamma }\right\}}^{\frac{1}{\gamma }}}\right),\\ \Delta \left(\tau -\frac{\tau }{1+{\left\{\phi {\left(\frac{\Delta^{-1}\left({ɇ}_{v},ℵ\right)}{\tau -\Delta^{-1}\left({ɇ}_{v},ℵ\right)}\right)}^{\gamma }\right\}}^{\frac{1}{\gamma }}}\right) \end{array}\right)$.

The article "A multiple attribute group decision making model based on 2-tuple linguistic pythagorean fuzzy dombi aggregation operators for optimal selection of potential global suppliers" was published in 2024. Journal: Heliyon.

The following lists several operations on 2TLPFNs that use the Dombi t−norm and Dombi t−conorm.

## 4 Dombi weighted aggregation operators with 2TLPFNs

This section introduces the 2TLPFDWAA and 2TLPFDWGA operators using the Dombi operational rules of 2TLPFNs. Moreover, certain important properties of these operators are investigated.

### 4.1 2-Tuple linguistic pythagorean fuzzy dombi arithematic aggregation operators

#### 4.1.1 Definition

Let ${¥}_{i}=\left(\left({ɇ}_{u_{i}},{£}_{i}\right),\left({ɇ}_{v_{i}},{ℵ}_{i}\right)\right),i=1,2,\ldots ,n)$ be the n number of 2TLPFNs. Then, Eq (11) presents that 2TLPFDWA operator is a function $f_{2TLPFDWA}^{w}:{¥}^{n}\to ¥$, such that,

$$f_{2TLPFDWA}^{w}\left({¥}_{1},{¥}_{2},\ldots ,{¥}_{n}\right)={⊕}_{i=1}^{n}\left(w_{i}{¥}_{i}\right)\text{.}$$

(11) $$f_{2TLPFDWA}^{w}\left({¥}_{1},{¥}_{2},\ldots ,{¥}_{n}\right)=\left(\begin{array}{c} \Delta \left(\tau \left(\sqrt[{2}]{1-\frac{1}{1+{\left\{\sum_{i=1}^{n}w_{i}{\left(\frac{{\left(\frac{\Delta^{-1}\left({ɇ}_{u_{i}},{£}_{i}\right)}{\tau }\right)}^{2}}{1-{\left(\frac{\Delta^{-1}\left({ɇ}_{u_{i}},{£}_{i}\right)}{\tau }\right)}^{2}}\right)}^{\gamma }\right\}}^{\frac{1}{\gamma }}}}\right)\right),\\ \Delta \left(\tau \left(\sqrt[{2}]{\frac{1}{1+{\left\{\sum_{i=1}^{n}w_{i}{\left(\frac{1-{\left(\frac{\Delta^{-1}\left({ɇ}_{v_{i}},{ℵ}_{i}\right)}{\tau }\right)}^{2}}{{\left(\frac{\Delta^{-1}\left({ɇ}_{v_{i}},{ℵ}_{i}\right)}{\tau }\right)}^{2}}\right)}^{\gamma }\right\}}^{\frac{1}{\gamma }}}}\right)\right) \end{array}\right)\text{.}$$

where, $w={\left(w_{1},w_{2},\ldots ,w_{n}\right)}^{T}$ be the weight vector of 2TLPFNs ${¥}_{i}$ for i=1,2,…,n, such that ${¥}_{i}>0$, γ≥1, and $\sum_{i=1}^{n}w_{i}=1$ for $w_{i}\in \left[0,1\right]$.

The article "A multiple attribute group decision making model based on 2-tuple linguistic pythagorean fuzzy dombi aggregation operators for optimal selection of potential global suppliers" was published in 2024. Journal: Heliyon.

Theorem 4.1.1 .

Let ${¥}_{i}=\left(\left({ɇ}_{u_{i}},{£}_{i}\right),\left({ɇ}_{v_{i}},{ℵ}_{i}\right)\right),i=1,2,\ldots ,n$ be the n number of 2TLPFNs for i=1,2,…,n, with the weight vector $w={\left(w_{1},w_{2},\ldots ,w_{n}\right)}^{T}$ of 2TLPFNs ${¥}_{i}>0$ for i=1,2,…,n, and $\sum_{i=1}^{n}w_{i}=1,\gamma \geq 1$.

$$f_{2TLPFDWA}^{w}\left({¥}_{1},{¥}_{2},\ldots ,{¥}_{n}\right)=\left(\begin{array}{c} \Delta \left(\tau \left(\sqrt[{2}]{1-\frac{1}{1+{\left\{\sum_{i=1}^{n}w_{i}{\left(\frac{{\left(\frac{\Delta^{-1}\left({ɇ}_{u_{i}},{£}_{i}\right)}{\tau }\right)}^{2}}{1-{\left(\frac{\Delta^{-1}\left({ɇ}_{u_{i}},{£}_{i}\right)}{\tau }\right)}^{2}}\right)}^{\gamma }\right\}}^{\frac{1}{\gamma }}}}\right)\right),\\ \Delta \left(\tau \left(\sqrt[{2}]{\frac{1}{1+{\left\{\sum_{i=1}^{n}w_{i}{\left(\frac{1-{\left(\frac{\Delta^{-1}\left({ɇ}_{v_{i}},{ℵ}_{i}\right)}{\tau }\right)}^{2}}{{\left(\frac{\Delta^{-1}\left({ɇ}_{v_{i}},{ℵ}_{i}\right)}{\tau }\right)}^{2}}\right)}^{\gamma }\right\}}^{\frac{1}{\gamma }}}}\right)\right) \end{array}\right)\text{.}$$

Proof:

For positive integer n, this theorem can be demonstrated by applying the inductive hypothesis.

If we take n=2. Then,

$$f_{2TLPFDWA}^{w}\left({¥}_{1},{¥}_{2}\right)=\left(\begin{array}{c} \Delta \left(\tau \left(\sqrt[{2}]{1-\frac{1}{1+{\left\{w_{1}{\left(\frac{{\left(\frac{\Delta^{-1}\left({ɇ}_{u_{1}},{£}_{1}\right)}{\tau }\right)}^{2}}{1-{\left(\frac{\Delta^{-1}\left({ɇ}_{u_{1}},{£}_{1}\right)}{\tau }\right)}^{2}}\right)}^{\gamma }+w_{2}{\left(\frac{{\left(\frac{\Delta^{-1}\left({ɇ}_{u_{2}},{£}_{2}\right)}{\tau }\right)}^{2}}{1-{\left(\frac{\Delta^{-1}\left({ɇ}_{u_{2}},{£}_{2}\right)}{\tau }\right)}^{2}}\right)}^{\gamma }\right\}}^{\frac{1}{\gamma }}}}\right)\right),\\ \Delta \left(\tau \left(\sqrt[{2}]{\frac{1}{1+{\left\{w_{1}{\left(\frac{1-{\left(\frac{\Delta^{-1}\left(\left({ɇ}_{v_{1}},{ℵ}_{1}\right)\right)}{\tau }\right)}^{2}}{{\left(\frac{\Delta^{-1}\left({ɇ}_{v_{1}},{ℵ}_{1}\right)}{\tau }\right)}^{2}}\right)}^{\gamma }+w_{2}{\left(\frac{1-{\left(\frac{\Delta^{-1}\left({ɇ}_{v_{2}},{ℵ}_{2}\right)}{\tau }\right)}^{2}}{{\left(\frac{\Delta^{-1}\left({ɇ}_{v_{2}},{ℵ}_{2}\right)}{\tau }\right)}^{2}}\right)}^{\gamma }\right\}}^{\frac{1}{\gamma }}}}\right)\right) \end{array}\right)\text{.}$$

$$=\left(\begin{array}{c} \Delta \left(\tau \left(\sqrt[{2}]{1-\frac{1}{1+{\left\{\sum_{i=1}^{2}w_{i}{\left(\frac{{\left(\frac{\Delta^{-1}\left({ɇ}_{u_{i}},{£}_{i}\right)}{\tau }\right)}^{2}}{1-{\left(\frac{\Delta^{-1}\left({ɇ}_{u_{i}},{£}_{i}\right)}{\tau }\right)}^{2}}\right)}^{\gamma }\right\}}^{\frac{1}{\gamma }}}}\right)\right),\\ \Delta \left(\tau \left(\sqrt[{2}]{\frac{1}{1+{\left\{\sum_{i=1}^{2}w_{i}{\left(\frac{1-{\left(\frac{\Delta^{-1}\left({ɇ}_{v_{i}},{ℵ}_{i}\right)}{\tau }\right)}^{2}}{{\left(\frac{\Delta^{-1}\left({ɇ}_{v_{i}},{ℵ}_{i}\right)}{\tau }\right)}^{2}}\right)}^{\gamma }\right\}}^{\frac{1}{\gamma }}}}\right)\right) \end{array}\right)\text{.}$$

For n=2, the theorem is therefore valid.

The article "A multiple attribute group decision making model based on 2-tuple linguistic pythagorean fuzzy dombi aggregation operators for optimal selection of potential global suppliers" was published in 2024. Journal: Heliyon.

Next, for s numbers of 2TLPFNs, we have

$$f_{2TLPFDWA}^{w}\left({¥}_{1},{¥}_{2},\ldots ,{¥}_{s}\right)={⊕}_{i=1}^{s}\left(w_{i}{¥}_{i}\right)\text{.}$$

Implies that,

$$f_{2TLPFDWA}^{w}\left({¥}_{1},{¥}_{2},\ldots ,{¥}_{s}\right)=\left(\begin{array}{c} \Delta \left(\tau \left(\sqrt[{2}]{1-\frac{1}{1+{\left\{\sum_{i=1}^{s}w_{i}{\left(\frac{{\left(\frac{\Delta^{-1}\left({ɇ}_{u_{i}},{£}_{i}\right)}{\tau }\right)}^{2}}{1-{\left(\frac{\Delta^{-1}\left({ɇ}_{u_{i}},{£}_{i}\right)}{\tau }\right)}^{2}}\right)}^{\gamma }\right\}}^{\frac{1}{\gamma }}}}\right)\right),\\ \Delta \left(\tau \left(\sqrt[{2}]{\frac{1}{1+{\left\{\sum_{i=1}^{s}w_{i}{\left(\frac{1-{\left(\frac{\Delta^{-1}\left({ɇ}_{v_{i}},{ℵ}_{i}\right)}{\tau }\right)}^{2}}{{\left(\frac{\Delta^{-1}\left({ɇ}_{v_{i}},{ℵ}_{i}\right)}{\tau }\right)}^{2}}\right)}^{\gamma }\right\}}^{\frac{1}{\gamma }}}}\right)\right) \end{array}\right)\text{.}$$

Now,

$$f_{2TLPFDWA}^{w}\left({¥}_{1},{¥}_{2},\ldots ,{¥}_{s},{¥}_{s+1}\right)={⊕}_{i=1}^{s+1}\left(w_{i}{¥}_{i}\right)={⊕}_{i=1}^{s}\left(w_{i}{¥}_{i}\right)⊕\left(w_{s+1}{¥}_{s+1}\right)\text{.}$$

$$=\left(\begin{array}{c} \Delta \left(\tau \left(\sqrt[{2}]{1-\frac{1}{1+{\left\{\sum_{i=1}^{s}w_{i}{\left(\frac{{\left(\frac{\Delta^{-1}\left({ɇ}_{u_{i}},{£}_{i}\right)}{\tau }\right)}^{2}}{1-{\left(\frac{\Delta^{-1}\left({ɇ}_{u_{i}},{£}_{i}\right)}{\tau }\right)}^{2}}\right)}^{\gamma }\right\}}^{\frac{1}{\gamma }}}}\right)\right),\\ \Delta \left(\tau \left(\sqrt[{2}]{\frac{1}{1+{\left\{\sum_{i=1}^{s}w_{i}{\left(\frac{1-{\left(\frac{\Delta^{-1}\left({ɇ}_{v_{i}},{ℵ}_{i}\right)}{\tau }\right)}^{2}}{{\left(\frac{\Delta^{-1}\left({ɇ}_{v_{i}},{ℵ}_{i}\right)}{\tau }\right)}^{2}}\right)}^{\gamma }\right\}}^{\frac{1}{\gamma }}}}\right)\right) \end{array}\right)⊕\left(\begin{array}{c} \Delta \left(\tau \left(\sqrt[{2}]{1-\frac{1}{1+{\left\{w_{s+1}{\left(\frac{{\left(\frac{\Delta^{-1}\left({ɇ}_{u_{s+1}},{£}_{s+1}\right)}{\tau }\right)}^{2}}{1-{\left(\frac{\Delta^{-1}\left({ɇ}_{u_{s+1}},{£}_{s+1}\right)}{\tau }\right)}^{2}}\right)}^{\gamma }\right\}}^{\frac{1}{\gamma }}}}\right)\right),\\ \Delta \left(\tau \left(\sqrt[{2}]{\frac{1}{1+{\left\{w_{s+1}{\left(\frac{1-{\left(\frac{\Delta^{-1}\left({ɇ}_{v_{s+1}},{ℵ}_{s+1}\right)}{\tau }\right)}^{2}}{{\left(\frac{\Delta^{-1}\left({ɇ}_{v_{s+1}},{ℵ}_{s+1}\right)}{\tau }\right)}^{2}}\right)}^{\gamma }\right\}}^{\frac{1}{\gamma }}}}\right)\right) \end{array}\right)\text{.}$$

$$=\left(\begin{array}{c} \Delta \left(\tau \left(\sqrt[{2}]{1-\frac{1}{1+{\left\{\sum_{i=1}^{s+1}w_{i}{\left(\frac{{\left(\frac{\Delta^{-1}\left({ɇ}_{u_{i}},{£}_{i}\right)}{\tau }\right)}^{2}}{1-{\left(\frac{\Delta^{-1}\left({ɇ}_{u_{i}},{£}_{i}\right)}{\tau }\right)}^{2}}\right)}^{\gamma }\right\}}^{\frac{1}{\gamma }}}}\right)\right),\\ \Delta \left(\tau \left(\sqrt[{2}]{\frac{1}{1+{\left\{\sum_{i=1}^{s+1}w_{i}{\left(\frac{1-{\left(\frac{\Delta^{-1}\left({ɇ}_{v_{i}},{ℵ}_{i}\right)}{\tau }\right)}^{2}}{{\left(\frac{\Delta^{-1}\left({ɇ}_{v_{i}},{ℵ}_{i}\right)}{\tau }\right)}^{2}}\right)}^{\gamma }\right\}}^{\frac{1}{\gamma }}}}\right)\right) \end{array}\right)\text{.}$$

Thus, the theorem is true for n=s+1. Thus, we determine that this assumption is accurate ∀n∈N.

The article "A multiple attribute group decision making model based on 2-tuple linguistic pythagorean fuzzy dombi aggregation operators for optimal selection of potential global suppliers" was published in 2024. Journal: Heliyon.

Theorem 4.1.2 .

(Idempotency property) Let ${¥}_{i}=\left(\left({ɇ}_{u_{i}},{£}_{i}\right),\left({ɇ}_{v_{i}},{ℵ}_{i}\right)\right)$ be the n 2TLPFNs for i=1,2,…,n. If the 2TLPFNs are all equal, that is, ${¥}_{i}=¥$ , ∀i. Then,

$$f_{2TLPFDWA}^{w}\left({¥}_{1},{¥}_{2},\ldots ,{¥}_{n}\right)=f_{2TLPFDWA}^{w}\left(¥,¥,\ldots ,¥\right)=¥=\left(\left({ɇ}_{u},£\right),\left({ɇ}_{v},ℵ\right)\right)\text{.}$$

Proof:

Let ${¥}_{i}=\left(\left({ɇ}_{u_{i}},{£}_{i}\right),\left({ɇ}_{v_{i}},{ℵ}_{i}\right)\right),i=1,2,\ldots ,n$ be the n 2TLPFNs which are all equal to $¥=\left(\left({ɇ}_{u},£\right),\left({ɇ}_{v},ℵ\right)\right)\text{.}$ Then,

$$f_{2TLPFDWA}^{w}\left({¥}_{1},{¥}_{2},\ldots ,{¥}_{n}\right)={⊕}_{i=1}^{n}\left(w_{i}{¥}_{i}\right)\text{.}$$

$$f_{2TLPFDWA}^{w}\left({¥}_{1},{¥}_{2},\ldots ,{¥}_{n}\right)=\left(\begin{array}{c} \Delta \left(\tau \left(\sqrt[{2}]{1-\frac{1}{1+{\left\{\sum_{i=1}^{n}w_{i}{\left(\frac{{\left(\frac{\Delta^{-1}\left({ɇ}_{u},£\right)}{\tau }\right)}^{2}}{1-{\left(\frac{\Delta^{-1}\left({ɇ}_{u},£\right)}{\tau }\right)}^{2}}\right)}^{\gamma }\right\}}^{\frac{1}{\gamma }}}}\right)\right),\\ \Delta \left(\tau \left(\sqrt[{2}]{\frac{1}{1+{\left\{\sum_{i=1}^{n}w_{i}{\left(\frac{1-{\left(\frac{\Delta^{-1}\left({ɇ}_{v},ℵ\right)}{\tau }\right)}^{2}}{{\left(\frac{\Delta^{-1}\left({ɇ}_{v},ℵ\right)}{\tau }\right)}^{2}}\right)}^{\gamma }\right\}}^{\frac{1}{\gamma }}}}\right)\right) \end{array}\right)\text{.}$$

$$=\left(\begin{array}{c} \Delta \left(\tau \left(\sqrt[{2}]{1-\frac{1}{1+{\left\{{\left(\frac{{\left(\frac{\Delta^{-1}\left({ɇ}_{u},£\right)}{\tau }\right)}^{2}}{1-{\left(\frac{\Delta^{-1}\left({ɇ}_{u},£\right)}{\tau }\right)}^{2}}\right)}^{\gamma }\right\}}^{\frac{1}{\gamma }}}}\right)\right),\\ \Delta \left(\tau \left(\sqrt[{2}]{\frac{1}{1+{\left\{{\left(\frac{1-{\left(\frac{\Delta^{-1}\left({ɇ}_{v},ℵ\right)}{\tau }\right)}^{2}}{{\left(\frac{\Delta^{-1}\left({ɇ}_{v},ℵ\right)}{\tau }\right)}^{2}}\right)}^{\gamma }\right\}}^{\frac{1}{\gamma }}}}\right)\right) \end{array}\right)\text{.}$$

$$=\left(\left({ɇ}_{u},£\right),\left({ɇ}_{v},ℵ\right)\right)=¥\text{.}$$

Hence the result is proved.

The article "A multiple attribute group decision making model based on 2-tuple linguistic pythagorean fuzzy dombi aggregation operators for optimal selection of potential global suppliers" was published in 2024. Journal: Heliyon.

Theorem 4.1.3 .

(Monotonicity property) Let ${¥}_{i}=\left(\left({ɇ}_{u_{i}},{£}_{i}\right),\left({ɇ}_{v_{i}},{ℵ}_{i}\right)\right)$ and ${{¥}_{i}}^{\prime }=\left(\left({{ɇ}_{u_{i}}}^{\prime },{{£}_{i}}^{\prime }\right),\left({{ɇ}_{v_{i}}}^{\prime },{{ℵ}_{i}}^{\prime }\right)\right)$ be two sets of 2TLPFNs, such that ${{¥}_{i}}^{\prime }\geq {¥}_{i}$ for i=1,2,…,n. Then,

$$f_{2TLPFDWA}^{w}\left({{¥}_{1}}^{\prime },{{¥}_{2}}^{\prime },\ldots ,{{¥}_{n}}^{\prime }\right)\geq f_{2TLPFDWA}^{w}\left({¥}_{1},{¥}_{2},\ldots ,{¥}_{n}\right)\text{.}$$

Proof:

Since, ${{¥}_{i}}^{\prime }\geq {¥}_{i}\text{,}$ then $\left({{ɇ}_{u_{i}}}^{\prime },{{£}_{i}}^{\prime }\right)\geq \left({ɇ}_{u_{i}},{£}_{i}\right)$ and $\left({{ɇ}_{v_{i}}}^{\prime },{{ℵ}_{i}}^{\prime }\right)\leq \left({ɇ}_{v_{i}},{ℵ}_{i}\right)$ for i=1,2,…,n.

(a) Let ${¥}_{i}=\left(\left({ɇ}_{u_{i}},{£}_{i}\right),\left({ɇ}_{v_{i}},{ℵ}_{i}\right)\right)$ and ${{¥}_{i}}^{\prime }=\left(\left({{ɇ}_{u_{i}}}^{\prime },{{£}_{i}}^{\prime }\right),\left({{ɇ}_{v_{i}}}^{\prime },{{ℵ}_{i}}^{\prime }\right)\right)$ for i=1,2,…,n.

Suppose that,

$$\left({{ɇ}_{u_{i}}}^{\prime },{{£}_{i}}^{\prime }\right)\geq \left({ɇ}_{u_{i}},{£}_{i}\right)\text{.}$$

Implies that,

$$\Delta^{-1}\left({{ɇ}_{u_{i}}}^{\prime },{{£}_{i}}^{\prime }\right)\geq \Delta^{-1}\left({ɇ}_{u_{i}},{£}_{i}\right)\text{.}$$

So,

$${\left(\frac{\Delta^{-1}\left({{ɇ}_{u_{i}}}^{\prime },{{£}_{i}}^{\prime }\right)}{\tau }\right)}^{2}\geq {\left(\frac{\Delta^{-1}\left({ɇ}_{u_{i}},{£}_{i}\right)}{\tau }\right)}^{2}\text{.}$$

We may obtain,

$$\left(\frac{{\left(\frac{\Delta^{-1}\left({{ɇ}_{u_{i}}}^{\prime },{{£}_{i}}^{\prime }\right)}{\tau }\right)}^{2}}{1-{\left(\frac{\Delta^{-1}\left({{ɇ}_{u_{i}}}^{\prime },{{£}_{i}}^{\prime }\right)}{\tau }\right)}^{2}}\right)\geq \left(\frac{{\left(\frac{\Delta^{-1}\left({ɇ}_{u_{i}},{£}_{i}\right)}{\tau }\right)}^{2}}{1-{\left(\frac{\Delta^{-1}\left({ɇ}_{u_{i}},{£}_{i}\right)}{\tau }\right)}^{2}}\right)\;\text{as}\;\Delta^{-1}\left({ɇ}_{u_{i}},{£}_{i}\right),\Delta^{-1}\left({{ɇ}_{u_{i}}}^{\prime },{{£}_{i}}^{\prime }\right)<\tau \text{.}$$

Also, for $w_{i}\in \left[0,1\right]$, γ>0, we have $,w_{i}{\left(\frac{{\left(\frac{\Delta^{-1}\left({{ɇ}_{u_{i}}}^{\prime },{{£}_{i}}^{\prime }\right)}{\tau }\right)}^{2}}{1-{\left(\frac{\Delta^{-1}\left({{ɇ}_{u_{i}}}^{\prime },{{£}_{i}}^{\prime }\right)}{\tau }\right)}^{2}}\right)}^{\gamma }{\geq w}_{i}{\left(\frac{{\left(\frac{\Delta^{-1}\left({ɇ}_{u_{i}},{£}_{i}\right)}{\tau }\right)}^{2}}{1-{\left(\frac{\Delta^{-1}\left({ɇ}_{u_{i}},{£}_{i}\right)}{\tau }\right)}^{2}}\right)}^{\gamma }\text{,}$ for any i.

$${1+\left\{\sum_{i=1}^{n}w_{i}{\left(\frac{{\left(\frac{\Delta^{-1}\left({{ɇ}_{u_{i}}}^{\prime },{{£}_{i}}^{\prime }\right)}{\tau }\right)}^{2}}{1-{\left(\frac{\Delta^{-1}\left({{ɇ}_{u_{i}}}^{\prime },{{£}_{i}}^{\prime }\right)}{\tau }\right)}^{2}}\right)}^{\gamma }\right\}}^{\frac{1}{\gamma }}\geq {1+\left\{\sum_{i=1}^{n}w_{i}{\left(\frac{{\left(\frac{\Delta^{-1}\left({ɇ}_{u_{i}},{£}_{i}\right)}{\tau }\right)}^{2}}{1-{\left(\frac{\Delta^{-1}\left({ɇ}_{u_{i}},{£}_{i}\right)}{\tau }\right)}^{2}}\right)}^{\gamma }\right\}}^{\frac{1}{\gamma }}\text{.}$$

$$\Rightarrow \left(\frac{1}{{1+\left\{\sum_{i=1}^{n}w_{i}{\left(\frac{{\left(\frac{\Delta^{-1}\left({{ɇ}_{u_{i}}}^{\prime },{{£}_{i}}^{\prime }\right)}{\tau }\right)}^{2}}{1-{\left(\frac{\Delta^{-1}\left({{ɇ}_{u_{i}}}^{\prime },{{£}_{i}}^{\prime }\right)}{\tau }\right)}^{2}}\right)}^{\gamma }\right\}}^{\frac{1}{\gamma }}}\right)\leq \left(\frac{1}{{1+\left\{\sum_{i=1}^{n}w_{i}{\left(\frac{{\left(\frac{\Delta^{-1}\left({ɇ}_{u_{i}},{£}_{i}\right)}{\tau }\right)}^{2}}{1-{\left(\frac{\Delta^{-1}\left({ɇ}_{u_{i}},{£}_{i}\right)}{\tau }\right)}^{2}}\right)}^{\gamma }\right\}}^{\frac{1}{\gamma }}}\right)\text{.}$$

$$\Rightarrow \left(1-\frac{1}{{1+\left\{\sum_{i=1}^{n}w_{i}{\left(\frac{{\left(\frac{\Delta^{-1}\left({{ɇ}_{u_{i}}}^{\prime },{{£}_{i}}^{\prime }\right)}{\tau }\right)}^{2}}{1-{\left(\frac{\Delta^{-1}\left({{ɇ}_{u_{i}}}^{\prime },{{£}_{i}}^{\prime }\right)}{\tau }\right)}^{2}}\right)}^{\gamma }\right\}}^{\frac{1}{\gamma }}}\right)\geq \left(1-\frac{1}{{1+\left\{\sum_{i=1}^{n}w_{i}{\left(\frac{{\left(\frac{\Delta^{-1}\left({ɇ}_{u_{i}},{£}_{i}\right)}{\tau }\right)}^{2}}{1-{\left(\frac{\Delta^{-1}\left({ɇ}_{u_{i}},{£}_{i}\right)}{\tau }\right)}^{2}}\right)}^{\gamma }\right\}}^{\frac{1}{\gamma }}}\right)\text{.}$$

$$\Rightarrow \tau \left(\sqrt[{2}]{1-\frac{1}{{1+\left\{\sum_{i=1}^{n}w_{i}{\left(\frac{{\left(\frac{\Delta^{-1}\left({{ɇ}_{u_{i}}}^{\prime },{{£}_{i}}^{\prime }\right)}{\tau }\right)}^{2}}{1-{\left(\frac{\Delta^{-1}\left({{ɇ}_{u_{i}}}^{\prime },{{£}_{i}}^{\prime }\right)}{\tau }\right)}^{2}}\right)}^{\gamma }\right\}}^{\frac{1}{\gamma }}}}\right)\geq \tau \left(\sqrt[{2}]{1-\frac{1}{{1+\left\{\sum_{i=1}^{n}w_{i}{\left(\frac{{\left(\frac{\Delta^{-1}\left({ɇ}_{u_{i}},{£}_{i}\right)}{\tau }\right)}^{2}}{1-{\left(\frac{\Delta^{-1}\left({ɇ}_{u_{i}},{£}_{i}\right)}{\tau }\right)}^{2}}\right)}^{\gamma }\right\}}^{\frac{1}{\gamma }}}}\right)\text{.}$$

$$\Rightarrow \Delta \left(\tau \left(\sqrt[{2}]{1-\frac{1}{{1+\left\{\sum_{i=1}^{n}w_{i}{\left(\frac{{\left(\frac{\Delta^{-1}\left({{ɇ}_{u_{i}}}^{\prime },{{£}_{i}}^{\prime }\right)}{\tau }\right)}^{2}}{1-{\left(\frac{\Delta^{-1}\left({{ɇ}_{u_{i}}}^{\prime },{{£}_{i}}^{\prime }\right)}{\tau }\right)}^{2}}\right)}^{\gamma }\right\}}^{\frac{1}{\gamma }}}}\right)\right)\geq \Delta \left(\tau \left(\sqrt[{2}]{1-\frac{1}{{1+\left\{\sum_{i=1}^{n}w_{i}{\left(\frac{{\left(\frac{\Delta^{-1}\left({ɇ}_{u_{i}},{£}_{i}\right)}{\tau }\right)}^{2}}{1-{\left(\frac{\Delta^{-1}\left({ɇ}_{u_{i}},{£}_{i}\right)}{\tau }\right)}^{2}}\right)}^{\gamma }\right\}}^{\frac{1}{\gamma }}}}\right)\right)\text{.}$$

(b) Again, we suppose that

$$\left({{ɇ}_{v_{i}}}^{\prime },{{ℵ}_{i}}^{\prime }\right)\leq \left({ɇ}_{v_{i}},{ℵ}_{i}\right)\text{.}$$

Implies that,

$$\Delta^{-1}\left({{ɇ}_{v_{i}}}^{\prime },{{ℵ}_{i}}^{\prime }\right)\leq \Delta^{-1}\left({ɇ}_{v_{i}},{ℵ}_{i}\right)\text{.}$$

$${\left(\frac{\Delta^{-1}\left({{ɇ}_{v_{i}}}^{\prime },{{ℵ}_{i}}^{\prime }\right)}{\tau }\right)}^{2}\leq {\left(\frac{\Delta^{-1}\left({ɇ}_{v_{i}},{ℵ}_{i}\right)}{\tau }\right)}^{2}\text{.}$$

So,

$$\frac{1-{\left(\frac{\Delta^{-1}\left({{ɇ}_{v_{i}}}^{\prime },{{ℵ}_{i}}^{\prime }\right)}{\tau }\right)}^{2}}{{\left(\frac{\Delta^{-1}\left({{ɇ}_{v_{i}}}^{\prime },{{ℵ}_{i}}^{\prime }\right)}{\tau }\right)}^{2}}\geq \frac{1-{\left(\frac{\Delta^{-1}\left({ɇ}_{v_{i}},{ℵ}_{i}\right)}{\tau }\right)}^{2}}{{\left(\frac{\Delta^{-1}\left({ɇ}_{v_{i}},{ℵ}_{i}\right)}{\tau }\right)}^{2}}\text{.}$$

Also, for $w_{i}\in \left[0,1\right]$, γ>0, implies that ${\;w}_{i}{\left(\frac{1-{\left(\frac{\Delta^{-1}\left({{ɇ}_{v_{i}}}^{\prime },{{ℵ}_{i}}^{\prime }\right)}{\tau }\right)}^{2}}{{\left(\frac{\Delta^{-1}\left({{ɇ}_{v_{i}}}^{\prime },{{ℵ}_{i}}^{\prime }\right)}{\tau }\right)}^{2}}\right)}^{\gamma }{\geq w}_{i}{\left(\frac{1-{\left(\frac{\Delta^{-1}\left({ɇ}_{v_{i}},{ℵ}_{i}\right)}{\tau }\right)}^{2}}{{\left(\frac{\Delta^{-1}\left({ɇ}_{v_{i}},{ℵ}_{i}\right)}{\tau }\right)}^{2}}\right)}^{\gamma }$ for any i.

The article "A multiple attribute group decision making model based on 2-tuple linguistic pythagorean fuzzy dombi aggregation operators for optimal selection of potential global suppliers" was published in 2024. Journal: Heliyon.

Now,

$${1+\left\{\sum_{i=1}^{n}{w_{i}\left(\frac{1-{\left(\frac{\Delta^{-1}\left({{ɇ}_{v_{i}}}^{\prime },{{ℵ}_{i}}^{\prime }\right)}{\tau }\right)}^{2}}{{\left(\frac{\Delta^{-1}\left({{ɇ}_{v_{i}}}^{\prime },{{ℵ}_{i}}^{\prime }\right)}{\tau }\right)}^{2}}\right)}^{\gamma }\right\}}^{\frac{1}{\gamma }}\geq {1+\left\{\sum_{i=1}^{n}w_{i}{\left(\frac{1-{\left(\frac{\Delta^{-1}\left({ɇ}_{v_{i}},{ℵ}_{i}\right)}{\tau }\right)}^{2}}{{\left(\frac{\Delta^{-1}\left({ɇ}_{v_{i}},{ℵ}_{i}\right)}{\tau }\right)}^{2}}\right)}^{\gamma }\right\}}^{\frac{1}{\gamma }}\text{.}$$

$$\Rightarrow \left(\frac{1}{{1+\left\{\sum_{i=1}^{n}{w_{i}\left(\frac{1-{\left(\frac{\Delta^{-1}\left({{ɇ}_{v_{i}}}^{\prime },{{ℵ}_{i}}^{\prime }\right)}{\tau }\right)}^{2}}{{\left(\frac{\Delta^{-1}\left({{ɇ}_{v_{i}}}^{\prime },{{ℵ}_{i}}^{\prime }\right)}{\tau }\right)}^{2}}\right)}^{\gamma }\right\}}^{\frac{1}{\gamma }}}\right)\leq \left(\frac{1}{{1+\left\{\sum_{i=1}^{n}w_{i}{\left(\frac{1-{\left(\frac{\Delta^{-1}\left({ɇ}_{v_{i}},{ℵ}_{i}\right)}{\tau }\right)}^{2}}{{\left(\frac{\Delta^{-1}\left({ɇ}_{v_{i}},{ℵ}_{i}\right)}{\tau }\right)}^{2}}\right)}^{\gamma }\right\}}^{\frac{1}{\gamma }}}\right)\text{.}$$

$$\Rightarrow \;\tau \left(\sqrt[{2}]{\frac{1}{{1+\left\{\sum_{i=1}^{n}{w_{i}\left(\frac{1-{\left(\frac{\Delta^{-1}\left({{ɇ}_{v_{i}}}^{\prime },{{ℵ}_{i}}^{\prime }\right)}{\tau }\right)}^{2}}{{\left(\frac{\Delta^{-1}\left({{ɇ}_{v_{i}}}^{\prime },{{ℵ}_{i}}^{\prime }\right)}{\tau }\right)}^{2}}\right)}^{\gamma }\right\}}^{\frac{1}{\gamma }}}}\right)\leq \tau \left(\sqrt[{2}]{\frac{1}{{1+\left\{\sum_{i=1}^{n}w_{i}{\left(\frac{1-{\left(\frac{\Delta^{-1}\left({ɇ}_{v_{i}},{ℵ}_{i}\right)}{\tau }\right)}^{2}}{{\left(\frac{\Delta^{-1}\left({ɇ}_{v_{i}},{ℵ}_{i}\right)}{\tau }\right)}^{2}}\right)}^{\gamma }\right\}}^{\frac{1}{\gamma }}}}\right)\text{.}$$

$$\Rightarrow \Delta \left(\tau \left(\sqrt[{2}]{\frac{1}{{1+\left\{\sum_{i=1}^{n}{w_{i}\left(\frac{1-{\left(\frac{\Delta^{-1}\left({{ɇ}_{v_{i}}}^{\prime },{{ℵ}_{i}}^{\prime }\right)}{\tau }\right)}^{2}}{{\left(\frac{\Delta^{-1}\left({{ɇ}_{v_{i}}}^{\prime },{{ℵ}_{i}}^{\prime }\right)}{\tau }\right)}^{2}}\right)}^{\gamma }\right\}}^{\frac{1}{\gamma }}}}\right)\right)\leq \Delta \left(\tau \left(\sqrt[{2}]{\frac{1}{{1+\left\{\sum_{i=1}^{n}w_{i}{\left(\frac{1-{\left(\frac{\Delta^{-1}\left({ɇ}_{v_{i}},{ℵ}_{i}\right)}{\tau }\right)}^{2}}{{\left(\frac{\Delta^{-1}\left({ɇ}_{v_{i}},{ℵ}_{i}\right)}{\tau }\right)}^{2}}\right)}^{\gamma }\right\}}^{\frac{1}{\gamma }}}}\right)\right)\text{.}$$

$$\Rightarrow \left(\begin{array}{c} \Delta \left(\tau \left(\sqrt[{2}]{1-\frac{1}{{1+\left\{\sum_{i=1}^{n}w_{i}{\left(\frac{{\left(\frac{\Delta^{-1}\left({{ɇ}_{u_{i}}}^{\prime },{{£}_{i}}^{\prime }\right)}{\tau }\right)}^{2}}{1-{\left(\frac{\Delta^{-1}\left({{ɇ}_{u_{i}}}^{\prime },{{£}_{i}}^{\prime }\right)}{\tau }\right)}^{2}}\right)}^{\gamma }\right\}}^{\frac{1}{\gamma }}}}\right)\right),\\ \Delta \left(\tau \left(\sqrt[{2}]{\frac{1}{{1+\left\{\sum_{i=1}^{n}{w_{i}\left(\frac{1-{\left(\frac{\Delta^{-1}\left({{ɇ}_{v_{i}}}^{\prime },{{ℵ}_{i}}^{\prime }\right)}{\tau }\right)}^{2}}{{\left(\frac{\Delta^{-1}\left({{ɇ}_{v_{i}}}^{\prime },{{ℵ}_{i}}^{\prime }\right)}{\tau }\right)}^{2}}\right)}^{\gamma }\right\}}^{\frac{1}{\gamma }}}}\right)\right) \end{array}\right)\geq \left(\begin{array}{c} \Delta \left(\tau \left(\sqrt[{2}]{1-\frac{1}{{1+\left\{\sum_{i=1}^{n}w_{i}{\left(\frac{{\left(\frac{\Delta^{-1}\left({ɇ}_{u_{i}},{£}_{i}\right)}{\tau }\right)}^{2}}{1-{\left(\frac{\Delta^{-1}\left({ɇ}_{u_{i}},{£}_{i}\right)}{\tau }\right)}^{2}}\right)}^{\gamma }\right\}}^{\frac{1}{\gamma }}}}\right)\right),\\ \Delta \left(\tau \left(\sqrt[{2}]{\frac{1}{{1+\left\{\sum_{i=1}^{n}w_{i}{\left(\frac{1-{\left(\frac{\Delta^{-1}\left({ɇ}_{v_{i}},{ℵ}_{i}\right)}{\tau }\right)}^{2}}{{\left(\frac{\Delta^{-1}\left({ɇ}_{v_{i}},{ℵ}_{i}\right)}{\tau }\right)}^{2}}\right)}^{\gamma }\right\}}^{\frac{1}{\gamma }}}}\right)\right) \end{array}\right)\text{.}$$

That is,

$$f_{2TLPFDWA}^{w}\left({{¥}_{1}}^{\prime },{{¥}_{2}}^{\prime },\ldots ,{{¥}_{n}}^{\prime }\right)\geq f_{2TLPFDWA}^{w}\left({¥}_{1},{¥}_{2},\ldots ,{¥}_{n}\right)\text{.}$$

Theorem 4.1.4 .

The article "A multiple attribute group decision making model based on 2-tuple linguistic pythagorean fuzzy dombi aggregation operators for optimal selection of potential global suppliers" was published in 2024. Journal: Heliyon.

(Boundedness property) Let ${¥}_{i}=\left(\left({ɇ}_{u_{i}},{£}_{i}\right),\left({ɇ}_{v_{i}},{ℵ}_{i}\right)\right)$ be the n number of 2TLPFNs for i=1,2,…,n. Then, the function $f_{2TLPFDWA}^{w}\left({¥}_{1},{¥}_{2},\ldots ,{¥}_{n}\right)$ is bounded. That is,

$$\left(\min_{i}\left({ɇ}_{u_{i}},{£}_{i}\right),\max_{i}\left({ɇ}_{v_{i}},{ℵ}_{i}\right)\right)\leq f_{2TLPFDWA}^{w}\left({¥}_{1},{¥}_{2},\ldots ,{¥}_{n}\right)\leq \left(\max_{i}\left({ɇ}_{u_{i}},{£}_{i}\right),\min_{i}\left({ɇ}_{v_{i}},{ℵ}_{i}\right)\right)\text{.}$$

Proof:

Since, $\min_{i}\left({ɇ}_{u_{i}},{£}_{i}\right)\leq \left({ɇ}_{u_{i}},{£}_{i}\right)\leq \max_{i}\left({ɇ}_{u_{i}},{£}_{i}\right)$ and $\max_{i}\left({ɇ}_{v_{i}},{ℵ}_{i}\right).\leq \left({ɇ}_{v_{i}},{ℵ}_{i}\right).\leq \min_{i}\left({ɇ}_{v_{i}},{ℵ}_{i}\right)$.

Then by monotonicity, we may derive

$$\left(\min_{i}\left({ɇ}_{u_{i}},{£}_{i}\right),\max_{i}\left({ɇ}_{v_{i}},{ℵ}_{i}\right)\right)\leq \left(\left({ɇ}_{u_{i}},{£}_{i}\right),\left({ɇ}_{v_{i}},{ℵ}_{i}\right)\right)\leq \left(\max_{i}\left({ɇ}_{u_{i}},{£}_{i}\right),\min_{i}\left({ɇ}_{v_{i}},{ℵ}_{i}\right)\right)\text{.}$$

Implies that,

$$\left(\min_{i}\left({ɇ}_{u_{i}},{£}_{i}\right),\max_{i}\left({ɇ}_{v_{i}},{ℵ}_{i}\right)\right)\leq f_{2TLPFDWA}^{w}\left({¥}_{1},{¥}_{2},\ldots ,{¥}_{n}\right)\leq \left(\max_{i}\left({ɇ}_{u_{i}},{£}_{i}\right),\min_{i}\left({ɇ}_{v_{i}},{ℵ}_{i}\right)\right)\text{.}$$

The article "A multiple attribute group decision making model based on 2-tuple linguistic pythagorean fuzzy dombi aggregation operators for optimal selection of potential global suppliers" was published in 2024. Journal: Heliyon.

#### 4.1.2 Definition 4.1.2

Let ${¥}_{i}=\left(\left({ɇ}_{u_{i}},{£}_{i}\right),\left({ɇ}_{v_{i}},{ℵ}_{i}\right)\right),i=1,2,\ldots ,n$ be the n number of 2TLPFNs. Then, Eq (12) presents that 2TLPFDOWA operator is a function $f_{2TLPFDOWA}^{w}:{¥}^{n}\to ¥$ such that,

$$f_{2TLPFDOWA}^{w}\left({¥}_{1},{¥}_{2},\ldots ,{¥}_{n}\right)={⊕}_{i=1}^{n}\left(w_{i}{¥}_{\left(i\right)}\right)\text{.}$$

(12) $$f_{2TLPFDOWA}^{w}\left({¥}_{1},{¥}_{2},\ldots ,{¥}_{n}\right)=\left(\begin{array}{c} \Delta \left(\tau \left(\sqrt[{2}]{1-\frac{1}{1+{\left\{\sum_{i=1}^{n}w_{i}{\left(\frac{{\left(\frac{\Delta^{-1}\left({ɇ}_{u_{\left(i\right)}},{£}_{\left(i\right)}\right)}{\tau }\right)}^{2}}{1-{\left(\frac{\Delta^{-1}\left({ɇ}_{u_{\left(i\right)}},{£}_{\left(i\right)}\right)}{\tau }\right)}^{2}}\right)}^{\gamma }\right\}}^{\frac{1}{\gamma }}}}\right)\right),\\ \Delta \left(\tau \left(\sqrt[{2}]{\frac{1}{1+{\left\{\sum_{i=1}^{n}w_{i}{\left(\frac{1-{\left(\frac{\Delta^{-1}\left({ɇ}_{v_{\left(i\right)}},{ℵ}_{\left(i\right)}\right)}{\tau }\right)}^{2}}{{\left(\frac{\Delta^{-1}\left({ɇ}_{v_{\left(i\right)}},{ℵ}_{\left(i\right)}\right)}{\tau }\right)}^{2}}\right)}^{\gamma }\right\}}^{\frac{1}{\gamma }}}}\right)\right) \end{array}\right)\text{.}$$

where, ${¥}_{\left(i\right)}=\left(\left({ɇ}_{u_{\left(i\right)}},{£}_{\left(i\right)}\right),\left({ɇ}_{v_{\left(i\right)}},{ℵ}_{\left(i\right)}\right)\right)$ is the ith largest of ${¥}_{1},{¥}_{2},\ldots ,{¥}_{n}\text{,}$ and $w={\left(w_{1},w_{2},\ldots ,w_{n}\right)}^{T}$ be the weight vector of 2TLPFNs ${¥}_{i}$ for i=1,2,…,n, such that ${¥}_{i}>0$, γ>0 and $\sum_{i=1}^{n}w_{i}=1$ for $w_{i}\in \left[0,1\right]$.

Theorem 4.1.5 .

(Idempotency property) Let ${¥}_{i}=\left(\left({ɇ}_{u_{i}},{£}_{i}\right),\left({ɇ}_{v_{i}},{ℵ}_{i}\right)\right)$ be the n number of 2TLPFNs for i=1,2,…,n. If the 2TLPFNs are all equal, that is, ${¥}_{i}=¥$ for all i. Then,

$$f_{2TLPFDOWA}^{w}\left({¥}_{1},{¥}_{2},\ldots ,{¥}_{n}\right)=f_{2TLPFDOWA}^{w}\left(¥,¥,\ldots ,¥\right)=¥=\left\{\left({ɇ}_{u},£\right),\left({ɇ}_{v},ℵ\right)\right\}\text{.}$$

Proof:

Proof is same as Theorem 4.1.2.

Theorem 4.1.6 .

(Monotonicity property) Let ${¥}_{i}=\left(\left({ɇ}_{u_{i}},{£}_{i}\right),\left({ɇ}_{v_{i}},{ℵ}_{i}\right)\right)$ and ${{¥}_{i}}^{\prime }=\left(\left({{ɇ}_{u_{i}}}^{\prime },{{£}_{i}}^{\prime }\right),\left({{ɇ}_{v_{i}}}^{\prime },{{ℵ}_{i}}^{\prime }\right)\right)$ be two sets of 2TLPFNs, satisfying ${{¥}_{i}}^{\prime }{¥}_{i}$ for i=1,2,…,n. Then,

$$f_{2TLPFDOWA}^{w}\left({{¥}_{1}}^{\prime },{{¥}_{2}}^{\prime },\ldots ,{{¥}_{n}}^{\prime }\right)\geq f_{2TLPFDOWA}^{w}\left({¥}_{1},{¥}_{2},\ldots ,{¥}_{n}\right)\text{.}$$

Proof:

Proof is same as Theorem 4.1.3.

The article "A multiple attribute group decision making model based on 2-tuple linguistic pythagorean fuzzy dombi aggregation operators for optimal selection of potential global suppliers" was published in 2024. Journal: Heliyon.

Theorem 4.1.7 .

(Boundedness property) Let ${¥}_{i}=\left(\left({ɇ}_{u_{i}},{£}_{i}\right),\left({ɇ}_{v_{i}},{ℵ}_{i}\right)\right)$ be the n 2TLPFNs for i=1,2,…,n. Then, the function $f_{2TLPFDOWA}^{w}\left({¥}_{1},{¥}_{2},\ldots ,{¥}_{n}\right)$ is bounded. That is,

$$\left(\min_{i}\left({ɇ}_{u_{i}},{£}_{i}\right),\max_{i}\left({ɇ}_{v_{i}},{ℵ}_{i}\right)\right)\leq f_{2TLPFDOWA}^{w}\left({¥}_{1},{¥}_{2},\ldots ,{¥}_{n}\right)\leq \left(\max_{i}\left({ɇ}_{u_{i}},{£}_{i}\right),\min_{i}\left({ɇ}_{v_{i}},{ℵ}_{i}\right)\right)\text{.}$$

Proof:

Proof is same as Theorem 4.1.4.

### 4.2 2-Tuple linguistic pythagorean fuzzy dombi Geometric Aggregation Operators

#### 4.2.1 Definition

Let ${¥}_{i}=\left(\left({ɇ}_{u_{i}},{£}_{i}\right),\left({ɇ}_{v_{i}},{ℵ}_{i}\right)\right),i=1,2,\ldots ,n$ be the n number of 2TLPFNs. Then, Eq (13) presents that 2TLPFDWG operator is a function $f_{2TLPFDWG}^{w}:{¥}^{n}\to ¥$, such that,

$$f_{2TLPFDWG}^{w}\left({¥}_{1},{¥}_{2},\ldots ,{¥}_{n}\right)={⊗}_{i=1}^{n}{\left({¥}_{i}\right)}^{w_{i}}\text{.}$$

(13) $$f_{2TLPFDWG}^{w}\left({¥}_{1},{¥}_{2},\ldots ,{¥}_{n}\right)=\left(\begin{array}{c} \Delta \left(\tau \left(\sqrt[{2}]{\frac{1}{1+{\left\{\sum_{i=1}^{n}w_{i}{\left(\frac{1-{\left(\frac{\Delta^{-1}\left({ɇ}_{u_{i}},{£}_{i}\right)}{\tau }\right)}^{2}}{{\left(\frac{\Delta^{-1}\left({ɇ}_{u_{i}},{£}_{i}\right)}{\tau }\right)}^{2}}\right)}^{\gamma }\right\}}^{\frac{1}{\gamma }}}}\right)\right),\\ \Delta \left(\tau \left(\sqrt[{2}]{1-\frac{1}{1+{\left\{\sum_{i=1}^{n}w_{i}{\left(\frac{{\left(\frac{\Delta^{-1}\left({ɇ}_{v_{i}},{ℵ}_{i}\right)}{\tau }\right)}^{2}}{1-{\left(\frac{\Delta^{-1}\left({ɇ}_{v_{i}},{ℵ}_{i}\right)}{\tau }\right)}^{2}}\right)}^{\gamma }\right\}}^{\frac{1}{\gamma }}}}\right)\right) \end{array}\right)\text{.}$$

where, $w={\left(w_{1},w_{2},\ldots ,w_{n}\right)}^{T}$ be the weight vector of 2TLPFNs ${¥}_{i}$ for i=1,2,…,n, such that ${¥}_{i}>0$, γ≥1 and $\sum_{i=1}^{n}w_{i}=1$ for $w_{i}\in \left[0,1\right]$.

Theorem 4.2.1 .

Let ${¥}_{i}=\left(\left({ɇ}_{u_{i}},{£}_{i}\right),\left({ɇ}_{v_{i}},{ℵ}_{i}\right)\right)$ be the n number of 2TLPFNs for i=1,2,…,n, with the weight vector $w={\left(w_{1},w_{2},\ldots ,w_{n}\right)}^{T}$ of 2TLPFNs ${¥}_{i}>0$ for i=1,2,…,n, and $\sum_{i=1}^{n}w_{i}=1,\gamma \geq 1$.

$$f_{2TLPFDWG}^{w}\left({¥}_{1},{¥}_{2},\ldots ,{¥}_{n}\right)=\left(\begin{array}{c} \Delta \left(\tau \left(\sqrt[{2}]{\frac{1}{1+{\left\{\sum_{i=1}^{n}w_{i}{\left(\frac{1-{\left(\frac{\Delta^{-1}\left({ɇ}_{u_{i}},{£}_{i}\right)}{\tau }\right)}^{2}}{{\left(\frac{\Delta^{-1}\left({ɇ}_{u_{i}},{£}_{i}\right)}{\tau }\right)}^{2}}\right)}^{\gamma }\right\}}^{\frac{1}{\gamma }}}}\right)\right),\\ \Delta \left(\tau \left(\sqrt[{2}]{1-\frac{1}{1+{\left\{\sum_{i=1}^{n}w_{i}{\left(\frac{{\left(\frac{\Delta^{-1}\left({ɇ}_{v_{i}},{ℵ}_{i}\right)}{\tau }\right)}^{2}}{1-{\left(\frac{\Delta^{-1}\left({ɇ}_{v_{i}},{ℵ}_{i}\right)}{\tau }\right)}^{2}}\right)}^{\gamma }\right\}}^{\frac{1}{\gamma }}}}\right)\right) \end{array}\right)\text{.}$$

Proof:

The proof is same as Theorem 4.1.1.

The article "A multiple attribute group decision making model based on 2-tuple linguistic pythagorean fuzzy dombi aggregation operators for optimal selection of potential global suppliers" was published in 2024. Journal: Heliyon.

Theorem 4.2.2 .

(Idempotency property) Let ${¥}_{i}=\left(\left({ɇ}_{u_{i}},{£}_{i}\right),\left({ɇ}_{v_{i}},{ℵ}_{i}\right)\right)$ be the n 2TLPFNs for i=1,2,…,n. If the 2TLPFNs are all equal, that is, ${¥}_{i}=¥$ , ∀i. Then,

$$f_{2TLPFDWG}^{w}\left({¥}_{1},{¥}_{2},\ldots ,{¥}_{n}\right)=f_{2TLPFDWG}^{w}\left(¥,¥,\ldots ,¥\right)=¥=\left(\left({ɇ}_{u},£\right),\left({ɇ}_{v},ℵ\right)\right)\text{.}$$

Proof:

The proof is same as Theorem 4.1.2.

Theorem 4.2.3 .

(Monotonicity property) Let ${¥}_{i}=\left(\left({ɇ}_{u_{i}},{£}_{i}\right),\left({ɇ}_{v_{i}},{ℵ}_{i}\right)\right)$ and ${{¥}_{i}}^{\prime }=\left(\left({{ɇ}_{u_{i}}}^{\prime },{{£}_{i}}^{\prime }\right),\left({{ɇ}_{v_{i}}}^{\prime },{{ℵ}_{i}}^{\prime }\right)\right)$ be two sets of 2TLPFNs, such that ${{¥}_{i}}^{\prime }\geq {¥}_{i}$ for i=1,2,…,n. Then,

$$f_{2TLPFDWG}^{w}\left({{¥}_{1}}^{\prime },{{¥}_{2}}^{\prime },\ldots ,{{¥}_{n}}^{\prime }\right)\geq f_{2TLPFDWG}^{w}\left({¥}_{1},{¥}_{2},\ldots ,{¥}_{n}\right)\text{.}$$

Proof:

The proof is same as Theorem 4.1.3.

Theorem 4.2.4 .

(Boundedness property) Let ${¥}_{i}=\left(\left({ɇ}_{u_{i}},{£}_{i}\right),\left({ɇ}_{v_{i}},{ℵ}_{i}\right)\right)$ be the n number of 2TLPFNs for i=1,2,…,n. Then, the function $f_{2TLPFDWG}^{w}\left({¥}_{1},{¥}_{2},\ldots ,{¥}_{n}\right)$ is bounded. That is,

$$\left(\min_{i}\left({ɇ}_{u_{i}},{£}_{i}\right),\max_{i}\left({ɇ}_{v_{i}},{ℵ}_{i}\right)\right)\leq f_{2TLPFDWG}^{w}\left({¥}_{1},{¥}_{2},\ldots ,{¥}_{n}\right)\leq \left(\max_{i}\left({ɇ}_{u_{i}},{£}_{i}\right),\min_{i}\left({ɇ}_{v_{i}},{ℵ}_{i}\right)\right)\text{.}$$

Proof:

The proof is same as Theorem 4.1.4.

#### 4.2.2 Definition

Let ${¥}_{i}=\left(\left({ɇ}_{u_{i}},{£}_{i}\right),\left({ɇ}_{v_{i}},{ℵ}_{i}\right)\right),i=1,2,\ldots ,n$ be the n number of 2TLPFNs. Then, Eq (14) presents that 2TLPFDOWG operator is a function $f_{2TLPFDOWG}^{w}:{¥}^{n}\to ¥$ such that,

$$f_{2TLPFDOWG}^{w}\left({¥}_{1},{¥}_{2},\ldots ,{¥}_{n}\right)={⊗}_{i=1}^{n}{\left({¥}_{\left(i\right)}\right)}^{w_{i}}\text{.}$$

(14) $$f_{2TLPFDOWG}^{w}\left({¥}_{1},{¥}_{2},\ldots ,{¥}_{n}\right)=\left(\begin{array}{c} \Delta \left(\tau \left(\sqrt[{2}]{\frac{1}{1+{\left\{\sum_{i=1}^{n}w_{i}{\left(\frac{1-{\left(\frac{\Delta^{-1}\left({ɇ}_{u_{\left(i\right)}},{£}_{\left(i\right)}\right)}{\tau }\right)}^{2}}{{\left(\frac{\Delta^{-1}\left({ɇ}_{u_{\left(i\right)}},{£}_{\left(i\right)}\right)}{\tau }\right)}^{2}}\right)}^{\gamma }\right\}}^{\frac{1}{\gamma }}}}\right)\right),\\ \Delta \left(\tau \left(\sqrt[{2}]{1-\frac{1}{1+{\left\{\sum_{i=1}^{n}w_{i}{\left(\frac{{\left(\frac{\Delta^{-1}\left({ɇ}_{v_{\left(i\right)}},{ℵ}_{\left(i\right)}\right)}{\tau }\right)}^{2}}{1-{\left(\frac{\Delta^{-1}\left({ɇ}_{v_{\left(i\right)}},{ℵ}_{\left(i\right)}\right)}{\tau }\right)}^{2}}\right)}^{\gamma }\right\}}^{\frac{1}{\gamma }}}}\right)\right) \end{array}\right)\text{.}$$

where, ${¥}_{\left(i\right)}=\left(\left({ɇ}_{u_{\left(i\right)}},{£}_{\left(i\right)}\right),\left({ɇ}_{v_{\left(i\right)}},{ℵ}_{\left(i\right)}\right)\right)$ is the ith largest of ${¥}_{1},{¥}_{2},\ldots ,{¥}_{n}\text{,}$ and $w={\left(w_{1},w_{2},\ldots ,w_{n}\right)}^{T}$ be the weight vector of 2TLPFNs ${¥}_{i}$ for i=1,2,…,n, such that ${¥}_{i}>0$, γ≥1 and $\sum_{i=1}^{n}w_{i}=1$ for $w_{i}\in \left[0,1\right]$.

The article "A multiple attribute group decision making model based on 2-tuple linguistic pythagorean fuzzy dombi aggregation operators for optimal selection of potential global suppliers" was published in 2024. Journal: Heliyon.

Theorem 4.2.5 .

(Idempotency property) Let ${¥}_{i}=\left(\left({ɇ}_{u_{i}},{£}_{i}\right),\left({ɇ}_{v_{i}},{ℵ}_{i}\right)\right)$ be the n number of 2TLPFNs for i=1,2,…,n. If the 2TLPFNs are all equal, that is, ${¥}_{i}=¥$ for all i. Then,

$$f_{2TLPFDOWG}^{w}\left({¥}_{1},{¥}_{2},\ldots ,{¥}_{n}\right)=f_{2TLPFDOWG}^{w}\left(¥,¥,\ldots ,¥\right)=¥=\left(\left({ɇ}_{u},£\right),\left({ɇ}_{v},ℵ\right)\right)\text{.}$$

Proof:

Proof is same as Theorem 4.1.2.

Theorem 4.2.6 .

(Monotonicity property) Let ${¥}_{i}=\left(\left({ɇ}_{u_{i}},{£}_{i}\right),\left({ɇ}_{v_{i}},{ℵ}_{i}\right)\right)$ and ${{¥}_{i}}^{\prime }=\left(\left({{ɇ}_{u_{i}}}^{\prime },{{£}_{i}}^{\prime }\right),\left({{ɇ}_{v_{i}}}^{\prime },{{ℵ}_{i}}^{\prime }\right)\right)$ be two sets of 2TLPFNs, satisfying ${{¥}_{i}}^{\prime }\geq {¥}_{i}$ for i=1,2,…,n. Then,

$$f_{2TLPFDOWG}^{w}\left({{¥}_{1}}^{\prime },{{¥}_{2}}^{\prime },\ldots ,{{¥}_{n}}^{\prime }\right)\geq f_{2TLPFDOWG}^{w}\left({¥}_{1},{¥}_{2},\ldots ,{¥}_{n}\right)\text{.}$$

Proof:

Proof is same as Theorem 4.1.3.

Theorem 4.2.7 .

(Boundedness property) Let ${¥}_{i}=\left(\left({ɇ}_{u_{i}},{£}_{i}\right),\left({ɇ}_{v_{i}},{ℵ}_{i}\right)\right)$ be the n 2TLPFNs for i=1,2,…,n. Then, the function $f_{2TLPFDOWG}^{w}\left({¥}_{1},{¥}_{2},\ldots ,{¥}_{n}\right)$ is bounded. That is,

$$\left(\min_{i}\left({ɇ}_{u_{i}},{£}_{i}\right),\max_{i}\left({ɇ}_{v_{i}},{ℵ}_{i}\right)\right)\leq f_{2TLPFDOWG}^{w}\left({¥}_{1},{¥}_{2},\ldots ,{¥}_{n}\right)\leq \left(\max_{i}\left({ɇ}_{u_{i}},{£}_{i}\right),\min_{i}\left({ɇ}_{v_{i}},{ℵ}_{i}\right)\right)\text{.}$$

Proof:

Proof is same as Theorem 4.1.4.

The article "A multiple attribute group decision making model based on 2-tuple linguistic pythagorean fuzzy dombi aggregation operators for optimal selection of potential global suppliers" was published in 2024. Journal: Heliyon.

## 5 Model for MAGDM problem using 2-tuple linguistic pythagorean fuzzy data

We will solve a MultipleAttributeGroupDecisionMaking(MAGDM) problem utilizing 2−TupleLinguistic PythagoreanFuzzyDombiaggregationoperators in this part. In this case, attribute values are represented as 2TLPFNs, while the corresponding weights of the 2TLPFNs are represented as actual numbers. Let $₪=\left\{{₪}_{1},{₪}_{2},\ldots ,{₪}_{m}\right\}$ denotes all alternatives, and $₹=\left\{{₹}_{1},{₹}_{2},\ldots ,{₹}_{n}\right\}$ denotes the set of all attributes, and the set $O=\left\{O_{1},O_{2},\ldots ,O_{z}\right\}$ represents all decision makers. Also, we have considered $w=\left(w_{1},w_{2},\ldots ,w_{n}\right)$ be the weights associated to the attributes satisfying $w_{j}>0$ for j=1,2,…,n and $\sum_{j=1}^{n}w_{j}=1$. We use 2TLPFNs ${¥}_{ij}^{k}=\left(\left({ɇ}_{u_{ij}}^{k},{£}_{ij}^{k}\right),\left({ɇ}_{v_{ij}}^{k},{ℵ}_{ij}^{k}\right)\right)$ as assessment values of alternatives ${₪}_{i}$ in correspondence to the attributes ${₹}_{j}$ by the decision makers $O_{k}$.

### 5.1 Procedure of 2-tuple linguistic pythagorean fuzzy decision making based on proposed operators

To get the best alternative, the proposed method is described as follows.

Step 1 Construct the 2TLPF decision matrix ${ᵹ}_{k}={\left({¥}_{ij}^{k}\right)}_{m\times n}$ and utilize the 2TLPFDOWA from Def. 4.1.2 and 2TLPFDOWG operator from Def. 4.2.2 to derive the decision matrix $ᵹ={\left({¥}_{ij}\right)}_{m\times n}$:

$${¥}_{ij}=\left(\left({ɇ}_{u_{ij}},{£}_{ij}\right),\left({ɇ}_{v_{ij}},{ℵ}_{ij}\right)\right)=f_{2TLPFDOWA}^{w}\left({¥}_{ij}^{1},{¥}_{ij}^{2},\ldots ,{¥}_{ij}^{z}\right)\text{.}$$

And

$${¥}_{ij}=\left(\left({ɇ}_{u_{ij}},{£}_{ij}\right),\left({ɇ}_{v_{ij}},{ℵ}_{ij}\right)\right)=f_{2TLPFDOWG}^{w}\left({¥}_{ij}^{1},{¥}_{ij}^{2},\ldots ,{¥}_{ij}^{z}\right)\text{.}$$

Step 2 Utilize 2TLPFDWA from Def. 4.1.1 and 2TLPFDWG operator from Def. 4.2.1 to derive the overall evaluation values ${¥}_{i}$ of the alternatives ${₪}_{i}\left(i=1,2,\ldots ,m\right)$.
Step 3 Determine the score values of overall evaluation values ${¥}_{i}\left(i=1,2,\ldots ,m\right)$ according to Def. 2.4.2 and choose the best alternative by ranking the score of evaluation values ${¥}_{i}$ of the alternatives ${₪}_{i}\left(i=1,2,\ldots ,m\right)$.

To further clarify the steps of the created MAGDM technique in this study, we provide the flowchart (Fig. 1).

**Fig. 1:** The flowchart of proposed magdm approach.

## 6 .Application of proposed MAGDM in supply chain management

Here, we adapted an example presented by Ref. [40] to choose the best potential global supplier with 2TLPFNs to demonstrate the proposed MAGDM model's MAGDM procedure. Consider a manufacturing company wants to choose the best supplier for its main goods. There are four possible potential global suppliers ${₪}_{i}\left(i=1,2,3,4\right)$ in SCM to select. The decision makes group uses five attributes to assess the four potential global suppliers:

1. ${₹}_{1}\;is\;the\;total\;product\;manufacturing\;cost\text{,}$
2. ${₹}_{2}\;is\;the\;production\;quality\text{,}$
3. ${₹}_{3}\;is\;the\;enteprise^{\prime }s\;service\;level\text{,}$
4. ${₹}_{4}\;is\;the\;enterprise^{\prime }s\;profile\text{,}$
5. ${₹}_{5}\;is\;the\;enterprise^{\prime }s\;risk$

The four potential global suppliers ${₪}_{i}\left(i=1,2,3,4\right)$ are to be evaluated with 2TLPFNs where, $w={\left(0.25,0.20,0.15,0.18,0.22\right)}^{T}$ is the attributes weighting vector, and $w={\left(0.25,0.30,0.20,0.25\right)}^{T}$ is the decision makers weighting vector. The decision makers use a predefined linguistic term set (LTS) $E=\left\{{ɇ}_{0}=extremely\;poor,{ɇ}_{1}=very\;poor,{ɇ}_{2}=poor,{ɇ}_{3}=slightly\;poor,{ɇ}_{4}=fair,{ɇ}_{5}=slightly\;good,{ɇ}_{6}=good,{ɇ}_{7}=very\;good,{ɇ}_{8}=extremely\;good\right\}$.

The article "A multiple attribute group decision making model based on 2-tuple linguistic pythagorean fuzzy dombi aggregation operators for optimal selection of potential global suppliers" was published in 2024. Journal: Heliyon.

To evaluate the potential global suppliers.

Now, by using the proposed method in this article, we'll find the desired supplier.

Step 1 The 2TLPFN decision matrices provided by the decision makers $O_{k}\left(k=1,2,3,4\right)$ are ${ᵹ}_{k}{=\left({¥}_{ij}^{k}\right)}_{4\times 5}\left(k=1,2,3,4\right)$, which are given in Table 2, Table 3, Table 4 and Table 5, respectively.

**Table 2:** Decision matrix (${ᵹ}_{1})$ of 2TLPFNs given by $O_{1}$.

	${₹}_{1}$	${₹}_{2}$	${₹}_{3}$	${₹}_{4}$	${₹}_{5}$
${₪}_{1}$	$\left(\begin{array}{c} \left({ɇ}_{7},0.\right)\text{,}\\ \left({ɇ}_{1},0.\right) \end{array}\right)$	$\left(\begin{array}{c} \left({ɇ}_{6},0.\right)\text{,}\\ \left({ɇ}_{2},0.\right) \end{array}\right)$	$\left(\begin{array}{c} \left({ɇ}_{4},0.\right)\text{,}\\ \left({ɇ}_{3},0.\right) \end{array}\right)$	$\left(\begin{array}{c} \left({ɇ}_{7},0.\right)\text{,}\\ \left({ɇ}_{1},0.\right) \end{array}\right)$	$\left(\begin{array}{c} \left({ɇ}_{5},0.\right)\text{,}\\ \left({ɇ}_{2},0.\right) \end{array}\right)$
${₪}_{2}$	$\left(\begin{array}{c} \left({ɇ}_{6},0.\right)\text{,}\\ \left({ɇ}_{2},0.\right) \end{array}\right)$	$\left(\begin{array}{c} \left({ɇ}_{5},0.\right)\text{,}\\ \left({ɇ}_{2},0.\right) \end{array}\right)$	$\left(\begin{array}{c} \left({ɇ}_{6},0.\right)\text{,}\\ \left({ɇ}_{1},0.\right) \end{array}\right)$	$\left(\begin{array}{c} \left({ɇ}_{6},0.\right)\text{,}\\ \left({ɇ}_{2},0.\right) \end{array}\right)$	$\left(\begin{array}{c} \left({ɇ}_{7},0.\right)\text{,}\\ \left({ɇ}_{1},0.\right) \end{array}\right)$
${₪}_{3}$	$\left(\begin{array}{c} \left({ɇ}_{6},0.\right)\text{,}\\ \left({ɇ}_{1},0.\right) \end{array}\right)$	$\left(\begin{array}{c} \left({ɇ}_{5},0.\right)\text{,}\\ \left({ɇ}_{3},0.\right) \end{array}\right)$	$\left(\begin{array}{c} \left({ɇ}_{7},0.\right)\text{,}\\ \left({ɇ}_{1},0.\right) \end{array}\right)$	$\left(\begin{array}{c} \left({ɇ}_{5},0.\right)\text{,}\\ \left({ɇ}_{1},0.\right) \end{array}\right)$	$\left(\begin{array}{c} \left({ɇ}_{3},0.\right)\text{,}\\ \left({ɇ}_{4},0.\right) \end{array}\right)$
${₪}_{4}$	$\left(\begin{array}{c} \left({ɇ}_{5},0.\right)\text{,}\\ \left({ɇ}_{2},0.\right) \end{array}\right)$	$\left(\begin{array}{c} \left({ɇ}_{7},0.\right)\text{,}\\ \left({ɇ}_{1},0.\right) \end{array}\right)$	$\left(\begin{array}{c} \left({ɇ}_{4},0.\right)\text{,}\\ \left({ɇ}_{3},0.\right) \end{array}\right)$	$\left(\begin{array}{c} \left({ɇ}_{6},0.\right)\text{,}\\ \left({ɇ}_{1},0.\right) \end{array}\right)$	$\left(\begin{array}{c} \left({ɇ}_{4},0.\right)\text{,}\\ \left({ɇ}_{4},0.\right) \end{array}\right)$

The article "A multiple attribute group decision making model based on 2-tuple linguistic pythagorean fuzzy dombi aggregation operators for optimal selection of potential global suppliers" was published in 2024. Journal: Heliyon.

**Table 3:** Decision matrix (${ᵹ}_{2})$ of 2TLPFNs given by $O_{2}$.

	${₹}_{1}$	${₹}_{2}$	${₹}_{3}$	${₹}_{4}$	${₹}_{5}$
${₪}_{1}$	$\left(\begin{array}{c} \left({ɇ}_{7},0.\right)\text{,}\\ \left({ɇ}_{1},0.\right) \end{array}\right)$	$\left(\begin{array}{c} \left({ɇ}_{4},0.\right)\text{,}\\ \left({ɇ}_{4},0.\right) \end{array}\right)$	$\left(\begin{array}{c} \left({ɇ}_{6},0.\right)\text{,}\\ \left({ɇ}_{2},0.\right) \end{array}\right)$	$\left(\begin{array}{c} \left({ɇ}_{5},0.\right)\text{,}\\ \left({ɇ}_{2},0.\right) \end{array}\right)$	$\left(\begin{array}{c} \left({ɇ}_{3},0.\right)\text{,}\\ \left({ɇ}_{5},0.\right) \end{array}\right)$
${₪}_{2}$	$\left(\begin{array}{c} \left({ɇ}_{7},0.\right)\text{,}\\ \left({ɇ}_{1},0.\right) \end{array}\right)$	$\left(\begin{array}{c} \left({ɇ}_{5},0.\right)\text{,}\\ \left({ɇ}_{1},0.\right) \end{array}\right)$	$\left(\begin{array}{c} \left({ɇ}_{6},0.\right)\text{,}\\ \left({ɇ}_{1},0.\right) \end{array}\right)$	$\left(\begin{array}{c} \left({ɇ}_{5},0.\right)\text{,}\\ \left({ɇ}_{2},0.\right) \end{array}\right)$	$\left(\begin{array}{c} \left({ɇ}_{4},0.\right)\text{,}\\ \left({ɇ}_{3},0.\right) \end{array}\right)$
${₪}_{3}$	$\left(\begin{array}{c} \left({ɇ}_{5},0.\right)\text{,}\\ \left({ɇ}_{2},0.\right) \end{array}\right)$	$\left(\begin{array}{c} \left({ɇ}_{6},0.\right)\text{,}\\ \left({ɇ}_{1},0.\right) \end{array}\right)$	$\left(\begin{array}{c} \left({ɇ}_{7},0.\right)\text{,}\\ \left({ɇ}_{1},0.\right) \end{array}\right)$	$\left(\begin{array}{c} \left({ɇ}_{5},0.\right)\text{,}\\ \left({ɇ}_{3},0.\right) \end{array}\right)$	$\left(\begin{array}{c} \left({ɇ}_{4},0.\right)\text{,}\\ \left({ɇ}_{4},0.\right) \end{array}\right)$
${₪}_{4}$	$\left(\begin{array}{c} \left({ɇ}_{6},0.\right)\text{,}\\ \left({ɇ}_{2},0.\right) \end{array}\right)$	$\left(\begin{array}{c} \left({ɇ}_{4},0.\right)\text{,}\\ \left({ɇ}_{3},0.\right) \end{array}\right)$	$\left(\begin{array}{c} \left({ɇ}_{5},0.\right)\text{,}\\ \left({ɇ}_{2},0.\right) \end{array}\right)$	$\left(\begin{array}{c} \left({ɇ}_{7},0.\right)\text{,}\\ \left({ɇ}_{1},0.\right) \end{array}\right)$	$\left(\begin{array}{c} \left({ɇ}_{5},0.\right)\text{,}\\ \left({ɇ}_{3},0.\right) \end{array}\right)$

The article "A multiple attribute group decision making model based on 2-tuple linguistic pythagorean fuzzy dombi aggregation operators for optimal selection of potential global suppliers" was published in 2024. Journal: Heliyon.

**Table 4:** Decision matrix (${ᵹ}_{3})$ of 2TLPFNs given by $O_{3}$.

	${₹}_{1}$	${₹}_{2}$	${₹}_{3}$	${₹}_{4}$	${₹}_{5}$
${₪}_{1}$	$\left(\begin{array}{c} \left({ɇ}_{6},0.\right)\text{,}\\ \left({ɇ}_{1},0.\right) \end{array}\right)$	$\left(\begin{array}{c} \left({ɇ}_{5},0.\right)\text{,}\\ \left({ɇ}_{2},0.\right) \end{array}\right)$	$\left(\begin{array}{c} \left({ɇ}_{3},0.\right)\text{,}\\ \left({ɇ}_{4},0.\right) \end{array}\right)$	$\left(\begin{array}{c} \left({ɇ}_{7},0.\right)\text{,}\\ \left({ɇ}_{1},0.\right) \end{array}\right)$	$\left(\begin{array}{c} \left({ɇ}_{5},0.\right)\text{,}\\ \left({ɇ}_{2},0.\right) \end{array}\right)$
${₪}_{2}$	$\left(\begin{array}{c} \left({ɇ}_{7},0.\right)\text{,}\\ \left({ɇ}_{1},0.\right) \end{array}\right)$	$\left(\begin{array}{c} \left({ɇ}_{6},0.\right)\text{,}\\ \left({ɇ}_{2},0.\right) \end{array}\right)$	$\left(\begin{array}{c} \left({ɇ}_{7},0.\right)\text{,}\\ \left({ɇ}_{1},0.\right) \end{array}\right)$	$\left(\begin{array}{c} \left({ɇ}_{6},0.\right)\text{,}\\ \left({ɇ}_{2},0.\right) \end{array}\right)$	$\left(\begin{array}{c} \left({ɇ}_{5},0.\right)\text{,}\\ \left({ɇ}_{1},0.\right) \end{array}\right)$
${₪}_{3}$	$\left(\begin{array}{c} \left({ɇ}_{6},0.\right)\text{,}\\ \left({ɇ}_{1},0.\right) \end{array}\right)$	$\left(\begin{array}{c} \left({ɇ}_{5},0.\right)\text{,}\\ \left({ɇ}_{3},0.\right) \end{array}\right)$	$\left(\begin{array}{c} \left({ɇ}_{7},0.\right)\text{,}\\ \left({ɇ}_{1},0.\right) \end{array}\right)$	$\left(\begin{array}{c} \left({ɇ}_{5},0.\right)\text{,}\\ \left({ɇ}_{1},0.\right) \end{array}\right)$	$\left(\begin{array}{c} \left({ɇ}_{3},0.\right)\text{,}\\ \left({ɇ}_{4},0.\right) \end{array}\right)$
${₪}_{4}$	$\left(\begin{array}{c} \left({ɇ}_{5},0.\right)\text{,}\\ \left({ɇ}_{2},0.\right) \end{array}\right)$	$\left(\begin{array}{c} \left({ɇ}_{7},0.\right)\text{,}\\ \left({ɇ}_{1},0.\right) \end{array}\right)$	$\left(\begin{array}{c} \left({ɇ}_{4},0.\right)\text{,}\\ \left({ɇ}_{3},0.\right) \end{array}\right)$	$\left(\begin{array}{c} \left({ɇ}_{6},0.\right)\text{,}\\ \left({ɇ}_{1},0.\right) \end{array}\right)$	$\left(\begin{array}{c} \left({ɇ}_{4},0.\right)\text{,}\\ \left({ɇ}_{4},0.\right) \end{array}\right)$

The article "A multiple attribute group decision making model based on 2-tuple linguistic pythagorean fuzzy dombi aggregation operators for optimal selection of potential global suppliers" was published in 2024. Journal: Heliyon.

**Table 5:** Decision matrix (${ᵹ}_{4})$ of 2TLPFNs given by $O_{4}$.

	${₹}_{1}$	${₹}_{2}$	${₹}_{3}$	${₹}_{4}$	${₹}_{5}$
${₪}_{1}$	$\left(\begin{array}{c} \left({ɇ}_{5},0.\right)\text{,}\\ \left({ɇ}_{3},0.\right) \end{array}\right)$	$\left(\begin{array}{c} \left({ɇ}_{4},0.\right)\text{,}\\ \left({ɇ}_{4},0.\right) \end{array}\right)$	$\left(\begin{array}{c} \left({ɇ}_{7},0.\right)\text{,}\\ \left({ɇ}_{1},0.\right) \end{array}\right)$	$\left(\begin{array}{c} \left({ɇ}_{5},0.\right)\text{,}\\ \left({ɇ}_{1},0.\right) \end{array}\right)$	$\left(\begin{array}{c} \left({ɇ}_{4},0.\right)\text{,}\\ \left({ɇ}_{2},0.\right) \end{array}\right)$
${₪}_{2}$	$\left(\begin{array}{c} \left({ɇ}_{6},0.\right)\text{,}\\ \left({ɇ}_{1},0.\right) \end{array}\right)$	$\left(\begin{array}{c} \left({ɇ}_{7},0.\right)\text{,}\\ \left({ɇ}_{1},0.\right) \end{array}\right)$	$\left(\begin{array}{c} \left({ɇ}_{6},0.\right)\text{,}\\ \left({ɇ}_{1},0.\right) \end{array}\right)$	$\left(\begin{array}{c} \left({ɇ}_{5},0.\right)\text{,}\\ \left({ɇ}_{2},0.\right) \end{array}\right)$	$\left(\begin{array}{c} \left({ɇ}_{6},0.\right)\text{,}\\ \left({ɇ}_{1},0.\right) \end{array}\right)$
${₪}_{3}$	$\left(\begin{array}{c} \left({ɇ}_{5},0.\right)\text{,}\\ \left({ɇ}_{2},0.\right) \end{array}\right)$	$\left(\begin{array}{c} \left({ɇ}_{3},0.\right)\text{,}\\ \left({ɇ}_{4},0.\right) \end{array}\right)$	$\left(\begin{array}{c} \left({ɇ}_{6},0.\right)\text{,}\\ \left({ɇ}_{2},0.\right) \end{array}\right)$	$\left(\begin{array}{c} \left({ɇ}_{3},0.\right)\text{,}\\ \left({ɇ}_{3},0.\right) \end{array}\right)$	$\left(\begin{array}{c} \left({ɇ}_{5},0.\right)\text{,}\\ \left({ɇ}_{2},0.\right) \end{array}\right)$
${₪}_{4}$	$\left(\begin{array}{c} \left({ɇ}_{4},0.\right)\text{,}\\ \left({ɇ}_{3},0.\right) \end{array}\right)$	$\left(\begin{array}{c} \left({ɇ}_{5},0.\right)\text{,}\\ \left({ɇ}_{1},0.\right) \end{array}\right)$	$\left(\begin{array}{c} \left({ɇ}_{4},0.\right)\text{,}\\ \left({ɇ}_{2},0.\right) \end{array}\right)$	$\left(\begin{array}{c} \left({ɇ}_{6},0.\right)\text{,}\\ \left({ɇ}_{2},0.\right) \end{array}\right)$	$\left(\begin{array}{c} \left({ɇ}_{5},0.\right)\text{,}\\ \left({ɇ}_{2},0.\right) \end{array}\right)$

Let $w=\left(w_{1},w_{2},w_{3},w_{4}\right)={\left(0.25,0.30,0.20,0.25\right)}^{T}$ be the expert weight vector. The aggregated decision matrix $ᵹ={\left({¥}_{ij}\right)}_{m\times n}$ obtained by using the 2TLPFDOWA operator is shown in Table 6, while the aggregated decision matrix $ᵹ={\left({¥}_{ij}\right)}_{m\times n}$ obtained by using the 2TLPFDOWG operator is shown in Table 7.

Step 2 Using the 2TLPFDWA operator, the overall assessment values ${¥}_{i}$ of ${₪}_{i}\left(i=1,2,3,4\right)$ with corresponding weight vector $w={\left(0.25,0.20,0.15,0.18,0.22\right)}^{T}$ are obtained, which is presented as:

$${¥}_{i}=f_{2TLPFDWA}^{w}\left({¥}_{i1},{¥}_{i2},{¥}_{i3},{¥}_{i4},{¥}_{i5}\right)\text{.}$$

The article "A multiple attribute group decision making model based on 2-tuple linguistic pythagorean fuzzy dombi aggregation operators for optimal selection of potential global suppliers" was published in 2024. Journal: Heliyon.

**Table 6:** The fused results by the 2TLPFDOWA operator.

	${₹}_{1}$	${₹}_{2}$	${₹}_{3}$	${₹}_{4}$	${₹}_{5}$
${₪}_{1}$	$\left(\begin{array}{c} \left({ɇ}_{7},-0.36016\right)\text{,}\\ \left({ɇ}_{1},0.13389\right) \end{array}\right)$	$\left(\begin{array}{c} \left({ɇ}_{5},0.05296\right)\text{,}\\ \left({ɇ}_{2},0.45718\right) \end{array}\right)$	$\left(\begin{array}{c} \left({ɇ}_{6},0.02444\right)\text{,}\\ \left({ɇ}_{2},-0.33989\right) \end{array}\right)$	$\left(\begin{array}{c} \left({ɇ}_{7},-0.42312\right)\text{,}\\ \left({ɇ}_{1},0.1094\right) \end{array}\right)$	$\left(\begin{array}{c} \left({ɇ}_{4},0.49094\right)\text{,}\\ \left({ɇ}_{2},0.25018\right) \end{array}\right)$
${₪}_{2}$	$\left(\begin{array}{c} \left({ɇ}_{7},-0.28894\right)\text{,}\\ \left({ɇ}_{1},0.1094\right) \end{array}\right)$	$\left(\begin{array}{c} \left({ɇ}_{6},0.18917\right)\text{,}\\ \left({ɇ}_{1},0.30466\right) \end{array}\right)$	$\left(\begin{array}{c} \left({ɇ}_{6},0.40205\right)\text{,}\\ \left({ɇ}_{1},0\right) \end{array}\right)$	$\left(\begin{array}{c} \left({ɇ}_{6},-0.34938\right)\text{,}\\ \left({ɇ}_{2},0\right) \end{array}\right)$	$\left(\begin{array}{c} \left({ɇ}_{6},0.12267\right)\text{,}\\ \left({ɇ}_{1},0.13389\right) \end{array}\right)$
${₪}_{3}$	$\left(\begin{array}{c} \left({ɇ}_{6},-0.34938\right)\text{,}\\ \left({ɇ}_{1},0.22859\right) \end{array}\right)$	$\left(\begin{array}{c} \left({ɇ}_{5},0.09601\right)\text{,}\\ \left({ɇ}_{2},-0.23548\right) \end{array}\right)$	$\left(\begin{array}{c} \left({ɇ}_{7},-0.14214\right)\text{,}\\ \left({ɇ}_{1},0.1094\right) \end{array}\right)$	$\left(\begin{array}{c} \left({ɇ}_{5},-0.31586\right)\text{,}\\ \left({ɇ}_{1},0.29099\right) \end{array}\right)$	$\left(\begin{array}{c} \left({ɇ}_{4},0.00252\right)\text{,}\\ \left({ɇ}_{3},0.02372\right) \end{array}\right)$
${₪}_{4}$	$\left(\begin{array}{c} \left({ɇ}_{5},0.18695\right)\text{,}\\ \left({ɇ}_{2},0.15526\right) \end{array}\right)$	$\left(\begin{array}{c} \left({ɇ}_{7},-0.46357\right)\text{,}\\ \left({ɇ}_{1},0.13389\right) \end{array}\right)$	$\left(\begin{array}{c} \left({ɇ}_{4},0.31488\right)\text{,}\\ \left({ɇ}_{2},0.3094\right) \end{array}\right)$	$\left(\begin{array}{c} \left({ɇ}_{6},0.40205\right)\text{,}\\ \left({ɇ}_{1},0.1094\right) \end{array}\right)$	$\left(\begin{array}{c} \left({ɇ}_{5},-0.37332\right)\text{,}\\ \left({ɇ}_{3},-0.15971\right) \end{array}\right)$

**Table 7:** The fused results by the 2TLPFDOWG operator.

	${₹}_{1}$	${₹}_{2}$	${₹}_{3}$	${₹}_{4}$	${₹}_{5}$
${₪}_{1}$	$\left(\begin{array}{c} \left({ɇ}_{6},0.11075\right)\text{,}\\ \left({ɇ}_{2},-0.20821\right) \end{array}\right)$	$\left(\begin{array}{c} \left({ɇ}_{5},-0.39075\right)\text{,}\\ \left({ɇ}_{3},0.17292\right) \end{array}\right)$	$\left(\begin{array}{c} \left({ɇ}_{4},0.31479\right)\text{,}\\ \left({ɇ}_{3},-0.19624\right) \end{array}\right)$	$\left(\begin{array}{c} \left({ɇ}_{6},-0.1504\right)\text{,}\\ \left({ɇ}_{1},0.33333\right) \end{array}\right)$	$\left(\begin{array}{c} \left({ɇ}_{4},0.00713\right)\text{,}\\ \left({ɇ}_{3},0.33446\right) \end{array}\right)$
${₪}_{2}$	$\left(\begin{array}{c} \left({ɇ}_{6},0.49234\right)\text{,}\\ \left({ɇ}_{1},0.33333\right) \end{array}\right)$	$\left(\begin{array}{c} \left({ɇ}_{6},-0.35985\right)\text{,}\\ \left({ɇ}_{2},-0.36106\right) \end{array}\right)$	$\left(\begin{array}{c} \left({ɇ}_{6},0.20946\right)\text{,}\\ \left({ɇ}_{1},0\right) \end{array}\right)$	$\left(\begin{array}{c} \left({ɇ}_{5},0.4818\right)\text{,}\\ \left({ɇ}_{2},0\right) \end{array}\right)$	$\left(\begin{array}{c} \left({ɇ}_{5},0.19452\right)\text{,}\\ \left({ɇ}_{2},-0.20821\right) \end{array}\right)$
${₪}_{3}$	$\left(\begin{array}{c} \left({ɇ}_{5},0.4818\right)\text{,}\\ \left({ɇ}_{2},-0.45523\right) \end{array}\right)$	$\left(\begin{array}{c} \left({ɇ}_{4},0.27482\right)\text{,}\\ \left({ɇ}_{3},0.04269\right) \end{array}\right)$	$\left(\begin{array}{c} \left({ɇ}_{7},-0.29607\right)\text{,}\\ \left({ɇ}_{1},0.33333\right) \end{array}\right)$	$\left(\begin{array}{c} \left({ɇ}_{4},0.16025\right)\text{,}\\ \left({ɇ}_{2},0.20688\right) \end{array}\right)$	$\left(\begin{array}{c} \left({ɇ}_{4},-0.43652\right)\text{,}\\ \left({ɇ}_{4},-0.32935\right) \end{array}\right)$
${₪}_{4}$	$\left(\begin{array}{c} \left({ɇ}_{5},-0.15325\right)\text{,}\\ \left({ɇ}_{2},0.3094\right) \end{array}\right)$	$\left(\begin{array}{c} \left({ɇ}_{5},0.35676\right)\text{,}\\ \left({ɇ}_{2},-0.20821\right) \end{array}\right)$	$\left(\begin{array}{c} \left({ɇ}_{4},0.19314\right)\text{,}\\ \left({ɇ}_{3},-0.47848\right) \end{array}\right)$	$\left(\begin{array}{c} \left({ɇ}_{6},0.20946\right)\text{,}\\ \left({ɇ}_{1},0.33333\right) \end{array}\right)$	$\left(\begin{array}{c} \left({ɇ}_{4},0.46656\right)\text{,}\\ \left({ɇ}_{3},0.37015\right) \end{array}\right)$

Now, with the help of Table 6, we have

$${¥}_{1}=\left(\begin{array}{c} \left({ɇ}_{6},0.07235\right),\\ \left({ɇ}_{1},0.45602\right) \end{array}\right)\text{.}$$

$${¥}_{2}=\left(\begin{array}{c} \left({ɇ}_{6},0.31217\right),\\ \left({ɇ}_{1},0.20672\right) \end{array}\right)\text{.}$$

$${¥}_{3}=\left(\begin{array}{c} \left({ɇ}_{6},-0.38853\right),\\ \left({ɇ}_{1},0.4377\right) \end{array}\right)\text{.}$$

$${¥}_{4}=\left(\begin{array}{c} \left({ɇ}_{6},-0.241\right),\\ \left({ɇ}_{2},-0.44021\right) \end{array}\right)\text{.}$$

Now, using the 2TLPFDWG operator, we can get the overall assessment values ${¥}_{i}$ of ${₪}_{i}\left(i=1,2,3,4\right)$ with the corresponding weight vector $w={\left(0.25,0.20,0.15,0.18,0.22\right)}^{T}$, which is given as:

$${¥}_{i}=f_{2TLPFDWG}^{w}\left({¥}_{i1},{¥}_{i2},{¥}_{i3},{¥}_{i4},{¥}_{i5}\right)\text{.}$$

Now, with the help of Table 7, we have

$${¥}_{1}=\left(\begin{array}{c} \left({ɇ}_{5},-0.1847\right),\\ \left({ɇ}_{3},-0.35297\right) \end{array}\right)\text{.}$$

$${\;¥}_{2}=\left(\begin{array}{c} \left({ɇ}_{6},-0.25057\right),\\ \left({ɇ}_{2},-0.39562\right) \end{array}\right)\text{.}$$

$${¥}_{3}=\left(\begin{array}{c} \left({ɇ}_{4},0.4576\right),\\ \left({ɇ}_{3},-0.36891\right) \end{array}\right)\text{.}$$

$${\;¥}_{4}=\left(\begin{array}{c} \left({ɇ}_{5},-0.11114\right),\\ \left({ɇ}_{2},0.43869\right) \end{array}\right)\text{.}$$

Step 3 Table 8 now displays the score values of ${¥}_{i}\left(i=1,2,3,4\right)$ using Def. 2.4.2 and 2TLPFDOWA and 2TLPFDWA operators.

The article "A multiple attribute group decision making model based on 2-tuple linguistic pythagorean fuzzy dombi aggregation operators for optimal selection of potential global suppliers" was published in 2024. Journal: Heliyon.

Table 9 now displays the score values of ${¥}_{i}\left(i=1,2,3,4\right)$ using Def. 2.4.2 and 2TLPFDOWG and 2TLPFDWG operators.

**Table 8:** Score values of ${¥}_{i}\left(i=1,2,3,4\right)$ obtained by utilizing 2TLPFDOWA and 2TLPFDWA operators.

	2TLPFDOWA 2TLPFDWA	Score values
${¥}_{1}$	$\left(\begin{array}{c} \left({ɇ}_{6},0.07235\right)\text{,}\\ \left({ɇ}_{1},0.45602\right) \end{array}\right)$	$\left({ɇ}_{6},0.17209\right)$
${¥}_{2}$	$\left(\begin{array}{c} \left({ɇ}_{6},0.31217\right)\text{,}\\ \left({ɇ}_{1},0.20672\right) \end{array}\right)$	$\left({ɇ}_{6},0.399207\right)$
${¥}_{3}$	$\left(\begin{array}{c} \left({ɇ}_{6},-0.38853\right)\text{,}\\ \left({ɇ}_{1},0.4377\right) \end{array}\right)$	$\left({ɇ}_{6},-0.161149\right)$
${¥}_{4}$	$\left(\begin{array}{c} \left({ɇ}_{6},-0.241\right)\text{,}\\ \left({ɇ}_{2},-0.44021\right) \end{array}\right)$	$\left({ɇ}_{6},-0.079179\right)$

**Table 9:** Score values of ${¥}_{i}\left(i=1,2,3,4\right)$ obtained by utilizing 2TLPFDOWG and 2TLPFDWG operators.

	2TLPFDOWG 2TLPFDWG	Scores values
${¥}_{1}$	$\left(\begin{array}{c} \left({ɇ}_{5},-0.1847\right)\text{,}\\ \left({ɇ}_{3},-0.35297\right) \end{array}\right)$	$\left({ɇ}_{5},0.011272\right)$
${¥}_{2}$	$\left(\begin{array}{c} \left({ɇ}_{6},-0.25057\right)\text{,}\\ \left({ɇ}_{2},-0.39562\right) \end{array}\right)$	$\left({ɇ}_{6},-0.094881\right)$
${¥}_{3}$	$\left(\begin{array}{c} \left({ɇ}_{4},0.4576\right)\text{,}\\ \left({ɇ}_{3},-0.36891\right) \end{array}\right)$	$\left({ɇ}_{5},-0.190777\right)$
${¥}_{4}$	$\left(\begin{array}{c} \left({ɇ}_{5},-0.11114\right)\text{,}\\ \left({ɇ}_{2},0.43869\right) \end{array}\right)$	$\left({ɇ}_{5},0.122109\right)$

The ranking of the alternatives is provided in Table 10 and Fig. 2, based on the score values of ${¥}_{i}\left(i=1,2,3,4\right)$ of alternatives ${₪}_{i}\left(1,2,3,4\right)$ by utilizing 2TLPFDOWA,2TLPFDWA,2TLPFDOWG, and 2TLPFDWG operators.

The article "A multiple attribute group decision making model based on 2-tuple linguistic pythagorean fuzzy dombi aggregation operators for optimal selection of potential global suppliers" was published in 2024. Journal: Heliyon.

**Table 10:** Ranking of the alternatives.

Operators Ranking	
2TLPFDOWA 2TLPFDWA	${₪}_{2}>{₪}_{1}>{₪}_{4}>{₪}_{3}$
2TLPFDOWG 2TLPFDWG	${₪}_{2}>{₪}_{4}>{₪}_{1}>{₪}_{3}$

**Fig. 2:** Ranking positions based on 2TLPFDOWA, 2TLPFDWA, 2TLPFDOWG, and 2TLPFDWG operators.

As a result of the above ranking, it is concluded that the potential global supplier $\left({₪}_{2}\right)$ is the best option.

### 6.1 Influence of parameter γ on final result

Table 11 and Table 12 exhibit the impacts of parameters in the 2TLPFDOWA, 2TLPFDWA, 2TLPFDOWG, and 2TLPFDWG operators to demonstrate the validity of the suggested approach in this study.

**Table 11:** Ranking results of different parameters for 2TLPFDOWA and 2TLPFDWA operators.

γ	Score Value ${€}_{s}\left({¥}_{i}\right)$	Ranking
1	${€}_{s}\left({¥}_{1}\right)=\left({ɇ}_{6},0.17209\right)$ ${€}_{s}\left({¥}_{2}\right)=\left({ɇ}_{6},0.399207\right)$ ${€}_{s}\left({¥}_{3}\right)=\left({ɇ}_{6},-0.161149\right)$ ${€}_{s}\left({¥}_{4}\right)=\left({ɇ}_{6},-0.079179\right)$	${₪}_{2}>{₪}_{1}>{₪}_{4}>{₪}_{3}$
2	${€}_{s}\left({¥}_{1}\right)=\left({ɇ}_{7},-0.398758\right)$ ${€}_{s}\left({¥}_{2}\right)=\left({ɇ}_{7},-0.432623\right)$ ${€}_{s}\left({¥}_{3}\right)=\left({ɇ}_{6},0.181661\right)$ ${€}_{s}\left({¥}_{4}\right)=\left({ɇ}_{6},0.266869\right)$	${₪}_{1}>{₪}_{2}>{₪}_{4}>{₪}_{3}$
3	${€}_{s}\left({¥}_{1}\right)=\left({ɇ}_{7},-0.356369\right)$ ${€}_{s}\left({¥}_{2}\right)=\left({ɇ}_{7},-0.320587\right)$ ${€}_{s}\left({¥}_{3}\right)=\left({ɇ}_{6},0.407529\right)$ ${€}_{s}\left({¥}_{4}\right)=\left({ɇ}_{6},0.482358\right)$	${₪}_{2}>{₪}_{1}>{₪}_{4}>{₪}_{3}$
4	${€}_{s}\left({¥}_{1}\right)=\left({ɇ}_{7},-0.266511\right)$ ${€}_{s}\left({¥}_{2}\right)=\left({ɇ}_{7},-0.247683\right)$ ${€}_{s}\left({¥}_{3}\right)=\left({ɇ}_{7},-0.449732\right)$ ${€}_{s}\left({¥}_{4}\right)=\left({ɇ}_{7},-0.389233\right)$	${₪}_{2}>{₪}_{1}>{₪}_{4}>{₪}_{3}$
5	${€}_{s}\left({¥}_{1}\right)=\left({ɇ}_{7},-0.211407\right)$ ${€}_{s}\left({¥}_{2}\right)=\left({ɇ}_{7},-0.199161\right)$ ${€}_{s}\left({¥}_{3}\right)=\left({ɇ}_{7},-0.357494\right)$ ${€}_{s}\left({¥}_{4}\right)=\left({ɇ}_{7},-0.308612\right)$	${₪}_{2}>{₪}_{1}>{₪}_{4}>{₪}_{3}$
6	${€}_{s}\left({¥}_{1}\right)=\left({ɇ}_{7},-0.174724\right)$ ${€}_{s}\left({¥}_{2}\right)=\left({ɇ}_{7},-0.165539\right)$ ${€}_{s}\left({¥}_{3}\right)=\left({ɇ}_{7},-0.294939\right)$ ${€}_{s}\left({¥}_{4}\right)=\left({ɇ}_{7},-0.254572\right)$	${₪}_{2}>{₪}_{1}>{₪}_{4}>{₪}_{3}$
7	${€}_{s}\left({¥}_{1}\right)=\left({ɇ}_{7},-0.148746\right)$ ${€}_{s}\left({¥}_{2}\right)=\left({ɇ}_{7},-0.141263\right)$ ${€}_{s}\left({¥}_{3}\right)=\left({ɇ}_{7},-0.25039\right)$ ${€}_{s}\left({¥}_{4}\right)=\left({ɇ}_{7},-0.216249\right)$	${₪}_{2}>{₪}_{1}>{₪}_{4}>{₪}_{3}$
8	${€}_{s}\left({¥}_{1}\right)=\left({ɇ}_{7},-0.129423\right)$ ${€}_{s}\left({¥}_{2}\right)=\left({ɇ}_{7},-0.123055\right)$ ${€}_{s}\left({¥}_{3}\right)=\left({ɇ}_{7},-0.217303\right)$ ${€}_{s}\left({¥}_{4}\right)=\left({ɇ}_{7},-0.18781\right)$	${₪}_{2}>{₪}_{1}>{₪}_{4}>{₪}_{3}$
9	${€}_{s}\left({¥}_{1}\right)=\left({ɇ}_{7},-0.114533\right)$ ${€}_{s}\left({¥}_{2}\right)=\left({ɇ}_{7},-0.10895\right)$ ${€}_{s}\left({¥}_{3}\right)=\left({ɇ}_{7},-0.191846\right)$ ${€}_{s}\left({¥}_{4}\right)=\left({ɇ}_{7},-0.165906\right)$	${₪}_{2}>{₪}_{1}>{₪}_{4}>{₪}_{3}$
10	${€}_{s}\left({¥}_{1}\right)=\left({ɇ}_{7},-0.102695\right)$ ${€}_{s}\left({¥}_{2}\right)=\left({ɇ}_{7},-0.097729\right)$ ${€}_{s}\left({¥}_{3}\right)=\left({ɇ}_{7},-0.171685\right)$ ${€}_{s}\left({¥}_{4}\right)=\left({ɇ}_{7},-0.14857\right)$	${₪}_{2}>{₪}_{1}>{₪}_{4}>{₪}_{3}$
100	${€}_{s}\left({¥}_{1}\right)=\left({ɇ}_{7},-0.009952\right)$ ${€}_{s}\left({¥}_{2}\right)=\left({ɇ}_{7},-0.009486\right)$ ${€}_{s}\left({¥}_{3}\right)=\left({ɇ}_{7},-0.016342\right)$ ${€}_{s}\left({¥}_{4}\right)=\left({ɇ}_{7},-0.01422\right)$	${₪}_{2}>{₪}_{1}>{₪}_{4}>{₪}_{3}$
1000	${€}_{s}\left({¥}_{1}\right)=\left({ɇ}_{7},-0.001007\right)$ ${€}_{s}\left({¥}_{2}\right)=\left({ɇ}_{7},-0.000959\right)$ ${€}_{s}\left({¥}_{3}\right)=\left({ɇ}_{7},-0.00163\right)$ ${€}_{s}\left({¥}_{4}\right)=\left({ɇ}_{7},-0.001424\right)$	${₪}_{2}>{₪}_{1}>{₪}_{4}>{₪}_{3}$

The article "A multiple attribute group decision making model based on 2-tuple linguistic pythagorean fuzzy dombi aggregation operators for optimal selection of potential global suppliers" was published in 2024. Journal: Heliyon.

**Table 12:** Ranking results for different parameters of 2TLPFDOWG and 2TLPFDWG operators.

γ	Score Value ${€}_{s}\left({¥}_{i}\right)$	Ranking
1	${€}_{s}\left({¥}_{1}\right)=\left({ɇ}_{5},0.011272\right)$ ${€}_{s}\left({¥}_{2}\right)=\left({ɇ}_{6},-0.094881\right)$ ${€}_{s}\left({¥}_{3}\right)=\left({ɇ}_{5},-0.190777\right)$ ${€}_{s}\left({¥}_{4}\right)=\left({ɇ}_{5},0.122109\right)$	${₪}_{2}>{₪}_{4}>{₪}_{1}>{₪}_{3}$
2	${€}_{s}\left({¥}_{1}\right)=\left({ɇ}_{4},0.497948\right)$ ${€}_{s}\left({¥}_{2}\right)=\left({ɇ}_{6},-0.351141\right)$ ${€}_{s}\left({¥}_{3}\right)=\left({ɇ}_{4},0.413043\right)$ ${€}_{s}\left({¥}_{4}\right)=\left({ɇ}_{5},-0.136097\right)$	${₪}_{2}>{₪}_{4}>{₪}_{1}>{₪}_{3}$
3	${€}_{s}\left({¥}_{1}\right)=\left({ɇ}_{4},0.150562\right)$ ${€}_{s}\left({¥}_{2}\right)=\left({ɇ}_{5},0.431261\right)$ ${€}_{s}\left({¥}_{3}\right)=\left({ɇ}_{4},0.179682\right)$ ${€}_{s}\left({¥}_{4}\right)=\left({ɇ}_{5},-0.313307\right)$	${₪}_{2}>{₪}_{4}>{₪}_{3}>{₪}_{1}$
4	${€}_{s}\left({¥}_{1}\right)=\left({ɇ}_{4},-0.081698\right)$ ${€}_{s}\left({¥}_{2}\right)=\left({ɇ}_{5},0.258569\right)$ ${€}_{s}\left({¥}_{3}\right)=\left({ɇ}_{4},0.039259\right)$ ${€}_{s}\left({¥}_{4}\right)=\left({ɇ}_{5},-0.438651\right)$	${₪}_{2}>{₪}_{4}>{₪}_{3}>{₪}_{1}$
5	${€}_{s}\left({¥}_{1}\right)=\left({ɇ}_{4},-0.242837\right)$ ${€}_{s}\left({¥}_{2}\right)=\left({ɇ}_{5},0.125398\right)$ ${€}_{s}\left({¥}_{3}\right)=\left({ɇ}_{4},-0.051496\right)$ ${€}_{s}\left({¥}_{4}\right)=\left({ɇ}_{4},0.470099\right)$	${₪}_{2}>{₪}_{4}>{₪}_{3}>{₪}_{1}$
6	${€}_{s}\left({¥}_{1}\right)=\left({ɇ}_{4},-0.359228\right)$ ${€}_{s}\left({¥}_{2}\right)=\left({ɇ}_{5},0.023602\right)$ ${€}_{s}\left({¥}_{3}\right)=\left({ɇ}_{4},-0.114138\right)$ ${€}_{s}\left({¥}_{4}\right)=\left({ɇ}_{4},0.401946\right)$	${₪}_{2}>{₪}_{4}>{₪}_{3}>{₪}_{1}$
7	${€}_{s}\left({¥}_{1}\right)=\left({ɇ}_{4},-0.446317\right)$ ${€}_{s}\left({¥}_{2}\right)=\left({ɇ}_{5},-0.054755\right)$ ${€}_{s}\left({¥}_{3}\right)=\left({ɇ}_{4},-0.159681\right)$ ${€}_{s}\left({¥}_{4}\right)=\left({ɇ}_{4},0.349811\right)$	${₪}_{2}>{₪}_{4}>{₪}_{3}>{₪}_{1}$
8	${€}_{s}\left({¥}_{1}\right)=\left({ɇ}_{3},0.486571\right)$ ${€}_{s}\left({¥}_{2}\right)=\left({ɇ}_{5},-0.115968\right)$ ${€}_{s}\left({¥}_{3}\right)=\left({ɇ}_{4},-0.194158\right)$ ${€}_{s}\left({¥}_{4}\right)=\left({ɇ}_{4},0.309021\right)$	${₪}_{2}>{₪}_{4}>{₪}_{3}>{₪}_{1}$
9	${€}_{s}\left({¥}_{1}\right)=\left({ɇ}_{3},0.43353\right)$ ${€}_{s}\left({¥}_{2}\right)=\left({ɇ}_{5},-0.164647\right)$ ${€}_{s}\left({¥}_{3}\right)=\left({ɇ}_{4},-0.221102\right)$ ${€}_{s}\left({¥}_{4}\right)=\left({ɇ}_{4},0.276432\right)$	${₪}_{2}>{₪}_{4}>{₪}_{3}>{₪}_{1}$
10	${€}_{s}\left({¥}_{1}\right)=\left({ɇ}_{3},0.390682\right)$ ${€}_{s}\left({¥}_{2}\right)=\left({ɇ}_{5},-0.20406\right)$ ${€}_{s}\left({¥}_{3}\right)=\left({ɇ}_{4},-0.242719\right)$ ${€}_{s}\left({¥}_{4}\right)=\left({ɇ}_{4},0.249915\right)$	${₪}_{2}>{₪}_{4}>{₪}_{3}>{₪}_{1}$
100	${€}_{s}\left({¥}_{1}\right)=\left({ɇ}_{3},0.039137\right)$ ${€}_{s}\left({¥}_{2}\right)=\left({ɇ}_{4},0.473283\right)$ ${€}_{s}\left({¥}_{3}\right)=\left({ɇ}_{4},-0.418044\right)$ ${€}_{s}\left({¥}_{4}\right)=\left({ɇ}_{4},0.025723\right)$	${₪}_{2}>{₪}_{4}>{₪}_{3}>{₪}_{1}$
1000	${€}_{s}\left({¥}_{1}\right)=\left({ɇ}_{3},0.00391\right)$ ${€}_{s}\left({¥}_{2}\right)=\left({ɇ}_{4},0.441074\right)$ ${€}_{s}\left({¥}_{3}\right)=\left({ɇ}_{4},-0.435554\right)$ ${€}_{s}\left({¥}_{4}\right)=\left({ɇ}_{4},0.002577\right)$	${₪}_{2}>{₪}_{4}>{₪}_{3}>{₪}_{1}$

Table 13 displays the ranking results for various parameters of 2TLPFDOWA, 2TLPFDWA, 2TLPFDOWG, and 2TLPFDWG operators.

The article "A multiple attribute group decision making model based on 2-tuple linguistic pythagorean fuzzy dombi aggregation operators for optimal selection of potential global suppliers" was published in 2024. Journal: Heliyon.

**Table 13:** Ranking results for different parameters of 2TLPFDOWA, 2TLPFDWA, 2TLPFDOWG, and 2TLPFDWG operators.

γ	2TLPFDOWA 2TLPFDWA	2TLPFDOWG 2TLPFDWG
1	${₪}_{2}>{₪}_{1}>{₪}_{4}>{₪}_{3}$	${₪}_{2}>{₪}_{4}>{₪}_{1}>{₪}_{3}$
2	${₪}_{1}>{₪}_{2}>{₪}_{4}>{₪}_{3}$	${₪}_{2}>{₪}_{4}>{₪}_{1}>{₪}_{3}$
3	${₪}_{2}>{₪}_{1}>{₪}_{4}>{₪}_{3}$	${₪}_{2}>{₪}_{4}>{₪}_{3}>{₪}_{1}$
4	${₪}_{2}>{₪}_{1}>{₪}_{4}>{₪}_{3}$	${₪}_{2}>{₪}_{4}>{₪}_{3}>{₪}_{1}$
5	${₪}_{2}>{₪}_{1}>{₪}_{4}>{₪}_{3}$	${₪}_{2}>{₪}_{4}>{₪}_{3}>{₪}_{1}$
6	${₪}_{2}>{₪}_{1}>{₪}_{4}>{₪}_{3}$	${₪}_{2}>{₪}_{4}>{₪}_{3}>{₪}_{1}$
7	${₪}_{2}>{₪}_{1}>{₪}_{4}>{₪}_{3}$	${₪}_{2}>{₪}_{4}>{₪}_{3}>{₪}_{1}$
8	${₪}_{2}>{₪}_{1}>{₪}_{4}>{₪}_{3}$	${₪}_{2}>{₪}_{4}>{₪}_{3}>{₪}_{1}$
9	${₪}_{2}>{₪}_{1}>{₪}_{4}>{₪}_{3}$	${₪}_{2}>{₪}_{4}>{₪}_{3}>{₪}_{1}$
10	${₪}_{2}>{₪}_{1}>{₪}_{4}>{₪}_{3}$	${₪}_{2}>{₪}_{4}>{₪}_{3}>{₪}_{1}$
100	${₪}_{2}>{₪}_{1}>{₪}_{4}>{₪}_{3}$	${₪}_{2}>{₪}_{4}>{₪}_{3}>{₪}_{1}$
1000	${₪}_{2}>{₪}_{1}>{₪}_{4}>{₪}_{3}$	${₪}_{2}>{₪}_{4}>{₪}_{3}>{₪}_{1}$

In this context of decision-making, the ranking orders generated by the 2TLPFDOWA, 2TLPFDWA, 2TLPFDOWGand2TLPFDWG operators display outstanding consistency, as shown in Table 13. The results of the suggested MAGDM technique for selecting green suppliers show that, while different values affect order ranking, the best choice remains constant.

The scores generated by applying the 2TLPFDOWA and 2TLPFDWA operators to the alternatives ${₪}_{i}\left(i=1,2,3,4\right)$ show differences that correspond to various values of the parameter γ. Fig. 3 depicts a graph with score values and matching γ values varying from 1 to 1000. It is clear that ${₪}_{4}\text{and}\;{₪}_{3}$ consistently maintain their third and fourth positions. However, at γ=2, ${₪}_{2}\text{and}$ ${₪}_{1}$ switched from first to second place, respectively. However, for every γ∈[1,1000], except at γ=2, ${₪}_{2}$ and ${₪}_{1}$ remain in first and second place, respectively.

**Fig. 3:** Score of the alternatives ${₪}_{i}\left(i=1,2,3,4\right)$ based on the 2TLPFDOWA and 2TLPFDWA operators whenγ∈[1,1000].

Using the 2TLPFDOWG and 2TLPFDWG operators, the generated score values show changes according to different values of the parameter γ for the alternatives ${₪}_{i}\left(i=1,2,3,4\right)$. Fig. 4 shows a graph of score values with associated γ values varying from 1 to 1000, and it can be seen that ${₪}_{2}\text{and}\;{₪}_{4}$ constantly hold their top and second place positions. However, at γ=3, ${₪}_{1}\text{and}\;{₪}_{3}$ moved from third to fourth place, respectively, and they hold their places after γ=3.

**Fig. 4:** Score of the alternatives ${₪}_{i}\left(i=1,2,3,4\right)$ based on the 2TLPFDOWG and 2TLPFDWG operators when γ∈[1,1000].

The article "A multiple attribute group decision making model based on 2-tuple linguistic pythagorean fuzzy dombi aggregation operators for optimal selection of potential global suppliers" was published in 2024. Journal: Heliyon.

### 6.2 Comparative analysis

We contrast our technique with the 2TLIFWA and 2TLIFWG operators [41], 2TLPFWA and 2TLPFWG operators [27]. It may appear that these operators are unconcerned with their relationship. Our suggested operators take into account the link between the arguments being aggregated. The suggested aggregation operators may consider not only the best aggregation but also prevent information loss during the aggregation process. The comparative results are listed in Table 14, and outlined graphically in Fig. 5. Such findings demonstrate the efficacy of the recommended operators and methodology.

**Table 14:** Comparison of proposed method with different approaches.

Operators	Score Values ${Ӎ}_{s}\left({Ɽ}_{i}\right)$	Ranking	Optimal Alternatives
2TLIFOWA 2TLIFWA [41]	${€}_{s}\left({¥}_{1}\right)=\left({ɇ}_{6},-0.079735\right)$ ${€}_{s}\left({¥}_{2}\right)=\left({ɇ}_{6},0.38832\right)$ ${€}_{s}\left({¥}_{3}\right)=\left({ɇ}_{6},-0.308985\right)$ ${€}_{s}\left({¥}_{4}\right)=\left({ɇ}_{6},-0.117575\right)$	${₪}_{2}>{₪}_{1}>{₪}_{4}>{₪}_{3}$	${₪}_{2}$
2TLIFOWG 2TLIFWG [41]	${€}_{s}\left({¥}_{1}\right)=\left({ɇ}_{5},0.438785\right)$ ${€}_{s}\left({¥}_{2}\right)=\left({ɇ}_{6},0.199595\right)$ ${€}_{s}\left({¥}_{3}\right)=\left({ɇ}_{5},0.243185\right)$ ${€}_{s}\left({¥}_{4}\right)=\left({ɇ}_{5},0.41929\right)$	${₪}_{2}>{₪}_{1}>{₪}_{4}>{₪}_{3}$	${₪}_{2}$
2TLPFOWA 2TLPFWA [27]	${€}_{s}\left({¥}_{1}\right)=\left({ɇ}_{6},-0.125672\right)$ ${€}_{s}\left({¥}_{2}\right)=\left({ɇ}_{6},0.259655\right)$ ${€}_{s}\left({¥}_{3}\right)=\left({ɇ}_{6},-0.426233\right)$ ${€}_{s}\left({¥}_{4}\right)=\left({ɇ}_{6},-0.341639\right)$	${₪}_{2}>{₪}_{1}>{₪}_{4}>{₪}_{3}$	${₪}_{2}$
2TLPFOWG 2TLPFWG [27]	${€}_{s}\left({¥}_{1}\right)=\left({ɇ}_{5},0.268575\right)$ ${€}_{s}\left({¥}_{2}\right)=\left({ɇ}_{6},0.010531\right)$ ${€}_{s}\left({¥}_{3}\right)=\left({ɇ}_{5},0.044659\right)$ ${€}_{s}\left({¥}_{4}\right)=\left({ɇ}_{5},0.253528\right)$	${₪}_{2}>{₪}_{1}>{₪}_{4}>{₪}_{3}$	${₪}_{2}$
2TLIFDOWA 2TLIFDWA	${€}_{s}\left({¥}_{1}\right)=\left({ɇ}_{6},0.216135\right)$ ${€}_{s}\left({¥}_{2}\right)=\left({ɇ}_{7},-0.482115\right)$ ${€}_{s}\left({¥}_{3}\right)=\left({ɇ}_{6},-0.01861\right)$ ${€}_{s}\left({¥}_{4}\right)=\left({ɇ}_{6},0.003345\right)$	${₪}_{2}>{₪}_{1}>{₪}_{4}>{₪}_{3}$	${₪}_{2}$
2TLIFDOWG 2TLIFDWG	${€}_{s}\left({¥}_{1}\right)=\left({ɇ}_{5},0.26235\right)$ ${€}_{s}\left({¥}_{2}\right)=\left({ɇ}_{6},0.1497\right)$ ${€}_{s}\left({¥}_{3}\right)=\left({ɇ}_{5},0.083665\right)$ ${€}_{s}\left({¥}_{4}\right)=\left({ɇ}_{5},0.32612\right)$	${₪}_{2}>{₪}_{4}>{₪}_{1}>{₪}_{3}$	${₪}_{2}$
2TLPFDOWA 2TLPFDWA (Proposed Operators)	${€}_{s}\left({¥}_{1}\right)=\left({ɇ}_{6},0.17209\right)$ ${€}_{s}\left({¥}_{2}\right)=\left({ɇ}_{6},0.399207\right)$ ${€}_{s}\left({¥}_{3}\right)=\left({ɇ}_{6},-0.161149\right)$ ${€}_{s}\left({¥}_{4}\right)=\left({ɇ}_{6},-0.079179\right)$	${₪}_{2}>{₪}_{1}>{₪}_{4}>{₪}_{3}$	${₪}_{2}$
2TLPFDOWG 2TLPFDWG (Proposed Operators)	${€}_{s}\left({¥}_{1}\right)=\left({ɇ}_{5},0.011272\right)$ ${€}_{s}\left({¥}_{2}\right)=\left({ɇ}_{6},-0.094881\right)$ ${€}_{s}\left({¥}_{3}\right)=\left({ɇ}_{5},-0.190777\right)$ ${€}_{s}\left({¥}_{4}\right)=\left({ɇ}_{5},0.122109\right)$	${₪}_{2}>{₪}_{4}>{₪}_{1}>{₪}_{3}$	${₪}_{2}$

The article "A multiple attribute group decision making model based on 2-tuple linguistic pythagorean fuzzy dombi aggregation operators for optimal selection of potential global suppliers" was published in 2024. Journal: Heliyon.

**Fig. 5:** Comparative analysis.

Furthermore, when compared to other authors' operators and techniques [27,41], our operators and methodology have significant capabilities. The findings are displayed in Fig. 6, Fig. 7, Fig. 8, respectively, which further demonstrates the validity of the approach suggested in this work using 2TLPFDW Averaging/Geometric aggregation operators by showing that all techniques have the same desirable alternative. The very useful aggregation operators for employing 2-Tuple Linguistic Pythagorean Fuzzy data in decision-making problems are 2TLPFDOWA, 2TLPFDWA, 2TLPFDOWG and 2TLPFDWG. As shown in Table 11, Table 12, the parameter γ indicates the decision makers’ inclinations, and the decision makers can select the appropriate value for γ based on their tendencies. By varying the value of the parameter γ, we can construct distinct scoring functions and thus distinct ranks for the alternative. Thus, when used with parameters, the established aggregation operators focus on providing us with more options and stability than the existing aggregation operators [27,41], since they enable us to have positive variations for the parameter focusing on various real-world situations, which would be an intriguing topic and one that merits additional research.

**Fig. 6:** Ranking positions based on 2TLIFOWA, 2TLIFWA, 2TLIFOWG, and 2TLIFWG operators.

**Fig. 7:** Ranking positions based on 2TLPFOWA, 2TLPFWA, 2TLPFOWG, and 2TLPFWG operators.

**Fig. 8:** Ranking positions based on 2TLIFDOWA, 2TLIFDWA, 2TLIFDOWG, and 2TLIFDWG operators.

## 7 Conclusions

This study introduces several novel operational laws for 2TLPFSs that depend on the Dombi t-norm and Dombi t-conorm. The operating laws are the basis for defining new aggregation operators, such as the 2TLPFDWA, 2TLPFDOWA, 2TLPFDWG, and 2TLPFDOWG operators. We analyze certain characteristics of the suggested operators. Furthermore, a technique has been developed to address MAGDM problems within the 2TLPF system, while also assessing these operators. The practicality and reliability of the methods have been demonstrated through a mathematical example. The application of our approach to solve the MAGDM problem is proven by the results produced through making use of the aggregation operators. We have demonstrated the advantages of our approach by conducting a comparative analysis with other renowned Multiple Attribute Group Decision Making (MAGDM) methodologies. Thus, this article has following limitations.

1. The proposed MAGDM technique appropriately depicts the wide range of the 2TLPF decision context. However, it is not able to implement when the combined square amount of MD and NMD is more than $\tau^{2}$.
2. The 2TLPFS can effectively handle ambiguous and unclear data, however it is unable to handle m-poler data.
3. Another issue in the technique is that the attribute values and weights for the criterion are mostly determined by expert judgment or may be fixed. As a result, human error may reduce the accuracy of the suggested technique's judgment.
4. Dombi t-norm and t-conorm are sensitive to parameter choice, computationally demanding, and can lack transparency in decision-making processes due to their complex nature.
5. The effectiveness of these operators can be compromised by inconsistent data. In practical MAGDM scenarios, data provided by different decision-makers may vary in quality, affecting the reliability of the aggregated results.

The article "A multiple attribute group decision making model based on 2-tuple linguistic pythagorean fuzzy dombi aggregation operators for optimal selection of potential global suppliers" was published in 2024. Journal: Heliyon.

The system of 2TLPF settings has numerous benefits, however occasionally they are unable to manage unpredictable information pertaining to human viewpoints. The decision-maker looks at resilient settings such as 2-Tuple Linguistic T-spherical fuzzy sets (2TLT-SFSs), 2-Tuple Linguistic Picture Fuzzy Sets (2TLPFSs), 2-Tuple Linguistic Fermatean Fuzzy Sets (2TLFFSs), 2-Tuple Linguistic q-Rung Orthopair Fuzzy Sets (2TLq-ROFSs) and 2-Tuple Linguistic Spherical Fuzzy Sets (2TLSFSs) in order to overcome this limitation. We strive to find solutions for challenging real-world problems in areas such as artificial intelligence, renewable energy, pattern recognition, and emerging technologies. The example data show that the method provides all three of the necessary features at the same time: it lessens the effects of biased values, it takes into account the correlations between attributes, and it surpasses the limitations of the current operational rules for 2TLPFSs. We plan to incorporate depth learning into the suggested aggregation processes and utilize them for text categorization and recommendation systems in the future. Our future plans involve implementing the proposed framework in various other areas, including smart e-tourism applications, bridge construction methods, residential place selection, handling large and diverse data sets from patients with multiple chronic diseases, real-time wearable health data sensors based on the Internet of Things (IoT), personalized social networking based on individual semantics, and biomass feedstock selection, among others. Further investigation is necessary to explore the expansion and use of 2TLPFNs in decision-making, risk analysis, and other domains characterized by uncertainty and fuzziness [[42], [43], [44], [45], [46], [47], [48], [49], [50], [51], [52]].

The article "A multiple attribute group decision making model based on 2-tuple linguistic pythagorean fuzzy dombi aggregation operators for optimal selection of potential global suppliers" was published in 2024. Journal: Heliyon.

## Data availability

All data generated or analyzed during this study are included in this published article (and its Supplementary Information files).

## CRediT authorship contribution statement

**Tmader Alballa:** Validation, Resources. **Ahmed Alamer:** Validation, Formal analysis, Data curation. **Khadija Nasir:** Writing – original draft, Validation, Methodology, Investigation, Formal analysis, Data curation, Conceptualization. **Awais Yousaf:** Validation, Supervision, Software, Conceptualization. **Somayah Abdualziz Alhabeeb:** Formal analysis, Data curation. **Hamiden Abd El-Wahed Khalifa:** Methodology, Investigation.

## Declaration of competing interest

The authors declare the following financial interests/personal relationships which may be considered as potential competing interests:Tmader Alballa reports article publishing charges was provided by Princess Nourah bint Abdulrahman University. Tmader Alballa reports a relationship with Princess Nourah bint Abdulrahman University that includes: employment and funding grants. If there are other authors, they declare that they have no known competing financial interests or personal relationships that could have appeared to influence the work reported in this paper.
